The article "N-Cubic q-Rung Orthopair Fuzzy Sets: Analysis of the Use of Mobile App in the Education Sector" was published in 2022. Journal: Comput Intell Neurosci.

# N-Cubic *q*-Rung Orthopair Fuzzy Sets: Analysis of the Use of Mobile App in the Education Sector

**DOI:** 10.1155/2022/9984314

**Published:** 2022-09-30

**Authors:** Joseph David Madasi, Salma Khan, Nasreen Kausar, Dragan Pamucar, Muhammad Gulistan, Ben Sorowen

**Affiliations:** ^1^College of Mathematics and Computer Science, Zhejiang Normal University, Zhejiang, China; ^2^Department of Mathematics and Statistics, Hazara University, Mansehra, Pakistan; ^3^Department of Mathematics, Faculty of Arts and Sciences, Yildiz Technical University, Esenler 34210, Istanbul, Turkey; ^4^Faculity of Organizational Sciences, University of Belgrade, Belgrade 11000, Serbia; ^5^Department of Mathematics and Statistics, Kyambogo University, P.O. Box 1, Kyambogo, Uganda

## Abstract

This study analyzes the description to examine the results of a new study and create the technique and also demonstrate the effectiveness of this technique. In this ever-changing world, students are increasingly encouraged to use mobile phones primarily to learn for educational purposes. The learning process is continuous and the goal has now been achieved. It has been replaced by online learning. Due to mobile phones as well as the many feature-oriented applications, students can study at their own place and use the application to spend their time understanding, because everything is accessible with a single click. To carry on the study we applied mobile applications for online education system. Now, because the traditional method is taken into consideration, it is normal to carry a bag full of books and copies and immerse yourself in the tradition of learning to write. However, it has been found that not all students learn when he takes notes. Therefore, we must make sure that the student focuses only on one thing at a time. To continue the research, we apply the N-cubic structure to q-rung orthopair fuzzy sets in multi-attribute group decision-making problems. This structure solves the problems of multi-attribute group decision-making techniques more generally.

## 1. Introduction

Decision-making is an empathic process that allows the selection of alternatives from a set of possible attributes. In decision-making problems the data were ambiguous and uncertain and the representation of data is no longer in real number. For this purpose many researchers developed different theories to handle such type of data. Among these researchers, Zadeh [1] developed the theme of fuzzy set (FS) theory that could determine uncertainty and vagueness in classic sets which are based on only two values logic 0 and 1. In 1975, Zadeh [2–4] further expanded his ideas to interval-valued fuzzy sets (IVFS). Atanassov [5, 6] later came up with the idea that using intuitionistic fuzzy sets (IFS) to assist with the significance of the membership value as well as the nonmembership value. Wang et al. [7] defined some interval-valued intuitionistic fuzzy aggregation operators with basic operations and properties. Intuitionistic fuzzy set was generalized to the Pythagorean fuzzy set (PFS) [8] which described the value of membership and nonmembership with the condition that the square sum is less or equal to 1. PFS was generalized to q-rung orthopair fuzzy set [9]. In 2018 Ali [10] defined a new type of q-rung orthopair fuzzy sets where the domain of the function defining a q-ROF set is the region made up of orbits. To deal with the decision information, Liu and Wang [11] proposed the q-rung orthopair fuzzy weighted averaging operator and the q-rung orthopair fuzzy weighted geometric operator. Wei et al. [12] presented q-rung orthopair fuzzy Maclaurin symmetric mean operators and their applications to potential evaluation of emerging technology commercialization. Many researchers [13, 14] used the different versions of q-rung orthopair fuzzy sets in different field such as q-rung orthopair fuzzy soft sets, q-rung orthopair fuzzy hypersoft sets, and their operators. In 2012, Jun et al. [15] combined FS and IVFS and developed the theme of cubic set. In decision-making theory aggregation operators is an important component. The conflicting criteria are included in the multi-attribute decision-making (MADM) task, and the conflicting criteria are aggregated to solve the problem [13, 16]. Most aggregation operators treat criteria on an individual basis; they do not take into account how criteria interact with each other or with common criteria. Kaur and Garg [17, 18] developed cubic intuitionistic fuzzy aggregation operators, which includes two components at the same time. One component provides the degree of membership in the form of an interval value for cubic intuitionistic fuzzy numbers (CIFNs), as well as the second component, gives the degree of nonmembership in the form of fuzzy values. Abbas et al. [19] have described a modified version in CIFS that is known informally as cubic Pythagorean fuzzy sets (CPFS). Zang et al. [20] generalized CPFS into cubic *q*-rung orthopair fuzzy sets (CqROFSs). This allows decision-makers to explain their ideas better in the context of a fuzzy environment. In 2009, Jun et al. [21] defined negative-valued functions as well as the N-structure. This paper is on BCK/BCI algebra as well as subtraction algebra. Rashid et al. [22] used the concept of the N-structure and developed the theme of N-cubic sets, aggregate operators, and other concepts related to it. In 2020, Petrovic and Kankaras [23] developed a hybridized IT2FS-DEMATEL-AHP-TOPSIS multicriteria decision-making approach for the selection and evaluation of criteria for determination of air traffic control radar position. Agarwal et al. [24] discussed the development of management tools and techniques in decision-making for policy makers which are based on scientific evidence. Ali et al. [25] developed Einstein geometric aggregation operators using complex interval-valued pythagorean fuzzy set with application in green supplier chain management. We are currently employing the N-structure concept for q-ROFSs. The Cq-ROFS is a database that describes IVqROFS and q-ROFS in a way that is related to uncertainty in the information. In order to demonstrate how this structure might be used in decision-making, we shall examine issues relating to the N-structure of cubic q-rung orthopair fuzzy sets in this article. Although this study can manage decision-making more efficiently than fuzzy sets, using it manually is not simple. Therefore, we must create computer programming in order to overcome these constraints. By merging the N-structure with cubic q-ROF sets, this structure more specifically overcame the uncertainty issues. N-cubic q-rung orthopair fuzzy sets can effectively capture expert evaluation data and minimize fuzziness in decision-making outcomes.

## 2. Materials and Methods

In this section we recall some basic materials and methods.

**Definition 1 (see [6]).**

Let $\hat{G}\neq$∅ be universal set, then q-ROFS $\hat{H}$ be defined as

(1) $$\begin{array}{c} \hat{H}=\left\{\langle \hat{g},{℧}_{\hat{H}}\left(\hat{g}\right),\Omega_{\hat{H}}\left(\hat{g}\right)|\hat{g}\in \hat{G}\rangle \right\}\text{,} \end{array}$$

where ${℧}_{\hat{H}}\left(\overset{´}{r}\right)$ and $\Omega_{\hat{H}}\left(\overset{´}{r}\right)$ are a mapping from $\hat{G}$ to [0,1], also satisfy the condition as

(2) $$\begin{array}{c} 0\leq {℧}_{\hat{H}}\leq 1,0\leq \Omega_{\hat{H}}\leq 1\text{,} \end{array}$$

and

(3) $$\begin{array}{c} 0\leq {\left({℧}_{\hat{H}}\left(\hat{g}\right)\right)}^{q}\leq 1,0\leq {\left(\Omega_{\hat{H}}\left(\hat{g}\right)\right)}^{q}\leq 1\text{,} \end{array}$$

where q ≥ 1 for all $\hat{g}\in \hat{G}$ and represent the membership degree and the nonmembership degree to set $\hat{H}$.

**Definition 2 (see [6]).**

Let $\hat{G}\neq$∅ be universal set, then (IVq-ROFS) $\hat{H}$ be defined as

(4) $$\begin{array}{c} \hat{H}=\left\{\langle \hat{g},{℧}_{\hat{H}}\left(\hat{g}\right),\Omega_{\hat{H}}\left(\hat{g}\right)|\hat{g}\in \hat{G}\rangle \right\}\text{,} \end{array}$$

where ${℧}_{\hat{H}}\left(\hat{g}\right)$ and $\Omega_{\hat{H}}\left(\hat{g}\right)$ are a mapping from $\hat{G}$ to [0,1],

(5) $$\begin{array}{c} {℧}_{P}\left(\hat{g}\right)=\left[{℧}_{\hat{H}}^{L}\left(\hat{g}\right),{℧}_{\hat{H}}^{U}\left(\hat{g}\right)\right]\text{,} \end{array}$$

and

(6) $$\begin{array}{c} \Omega_{\hat{H}}\left(\hat{g}\right)=\left[\Omega_{\hat{H}}^{L}\left(\hat{g}\right),\Omega_{\hat{H}}^{U}\left(\hat{g}\right)\right], \end{array}$$

also satisfy the condition as

(7) $$\begin{array}{c} 0\leq {℧}_{\hat{H}}\leq 1,0\leq \Omega_{\hat{H}}\leq 1\text{,} \end{array}$$

and

(8) $$\begin{array}{c} 0\leq {\left({℧}_{\hat{H}}^{U}\left(\hat{g}\right)\right)}^{q}\leq 1,0\leq {\left(\Omega_{\hat{H}}^{U}\left(\hat{g}\right)\right)}^{q}\leq 1\text{,} \end{array}$$

where q ≥ 1 for all $\hat{g}\in \hat{G}$ and represent the membership degree and the nonmembership degree to set $\hat{H}$.

**Definition 3 (see [10]).**

Let *X* be the collection of some elements. A cubic-q-rung orthopair fuzzy set is represented as C={〈x, H(x), *ϑ*(x)*|*x ∈ X〉}, where H(x) is an Interval-valued-q-rung orthopair fuzzy set and *ϑ*(x) is a q-rung orthopair fuzzy set. Here H(x)={[℧^L^, ℧^U^][Ω^L^, Ω^U^]} such that 0 ≤ (℧^U^)^q^+(Ω^U^)^q^ ≤ 1 and *ϑ*(x)=(℧, Ω) with 0 ≤ ℧^q^+Ω^q^ ≤ 1 where q ≥ 1. It can be described as C=〈H, *ϑ*〉, where H={[℧^L^, ℧^U^][Ω^L^, Ω^U^]} and *ϑ*(x)=(℧, Ω) and it is known as the cubic-q-rung orthopair fuzzy set number.

## 3. *N*-Cubic *q*-Rung Orthopair Fuzzy Set and Hamy Mean Operators

This part develops the Nq-ROFS and NIVq-ROFS structures and introduces the innovative NCq-ROFS structure. The NCq-ROFS's accuracy and score functions are defined. Both N-cubic q-rung orthopair fuzzy Hamy mean operator and N-cubic q-rung orthopair fuzzy power Hamy mean operator, as well as their characteristics and weighted forms, are covered in this section.

**Definition 4 .**

Let *X* be the collection of some elements. A Nq-ROFS define asN^QRO^={〈x, F_N^QRO^_(x), H_N^QRO^_(x)〉 : x ∈ X} such that $-1\leq {\left(-1\right)}^{2\overset{˘}{q}+1}\left({\left(F_{N^{QRO}}\right)}^{2\overset{˘}{q}}+{\left(H_{N^{QRO}}\right)}^{2\overset{˘}{q}}\right)\leq 0$, where F_N^QRO^_(x) : X⟶[−1,0] and H_N^QRO^_(x) : X⟶[−1,0].

**Definition 5 .**

A NIVq-ROFS in a *ϕ* ≠ X is define as

(9) $$\begin{array}{c} N^{IV-QRO}=\left\{\langle \begin{array}{c} x,{\tilde{℧}}_{N^{IV-QRO}}\left(x\right)=\left[{℧}_{N^{IV-QRO}}^{L},{℧}_{N^{IV-QRO}}^{U}\right],\\ {\tilde{\Omega }}_{N^{IV-QRO}}\left(x\right)=\left[\Omega_{N^{IV-QRO}}^{L},\Omega_{N^{IV-QRO}}^{U}\right] \end{array}\rangle :x\in x\right\}, \end{array}$$

with the condition

(10) $$\begin{array}{c} -1\leq {\left(-1\right)}^{2\overset{˘}{q}+1}\left({\left({℧}_{N^{CQRO}}^{U}\right)}^{2\overset{˘}{q}}+{\left(\Omega_{N^{CQRO}}^{U}\right)}^{2\overset{˘}{q}}\right)\leq 0\text{,} \end{array}$$

where [℧_N^IV−QRO^_^L^, ℧_N^IV−QRO^_^U^] : X⟶[−1,0] and [Ω_N^IV−QRO^_^L^, Ω_N^IV−QRO^_^U^] : X⟶[−1,0].

**Definition 6 .**

An NCq-ROFS in a *ϕ* ≠ X is define by the structure N^CQRO^ = {〈x, Γ_N^CQRO^_(x), Ϝ_N^CQRO^_(x)〉 : x ∈ X}, where $\Gamma_{N^{CQRO}}=\left\{\langle x,{\tilde{℧}}_{N^{CQRO}}\left(x\right),{\tilde{\Omega }}_{N^{CQRO}}\left(x\right)\rangle :x\in X\right\}$ is an N−IVQROFS and Ϝ_N^CQRO^_ = {〈x, F_N^CQRO^_(x), H_N^CQRO^_(x)〉 : x ∈ X} is an N−QROFS. Here Γ_N^CQRO^_ = {[℧_N^CQRO^_^L^, ℧_N^CQRO^_^U^], [Ω_N^CQRO^_^L^, Ω_N^CQRO^_^U^]} : X⟶D[−1,0] with the condition that$-1\leq {\left(-1\right)}^{2\overset{˘}{q}+1}\left({\left({℧}_{N^{CQRO}}^{U}\right)}^{2\overset{˘}{q}}+{\left(\Omega_{N^{CQRO}}^{U}\right)}^{2\overset{˘}{q}}\right)\leq 0$ and Ϝ_N^CQRO^_ = {F_N^CQRO^_, H_N^CQRO^_} : X⟶[−1,0] with the condition$-1\leq {\left(-1\right)}^{2\overset{˘}{q}+1}\left({\left(F_{N^{CQRO}}\right)}^{2\overset{˘}{q}}+{\left(H_{N^{CQRO}}\right)}^{2\overset{˘}{q}}\right)\leq 0$. For simplicity it is denoted by N^CQRO^ = 〈Γ_N^CQRO^_, Ϝ_N^CQRO^_〉.

**Definition 7 .**

An NCq-ROF set N^CQRO^ = 〈Γ_N^CQRO^_, Ϝ_N^CQRO^_〉 in *ϕ* ≠ X is called internal NCq-ROF set if F_N^CQRO^_ ∈ [℧_N^CQRO^_^L^, ℧_N^CQRO^_^U^] and H_N^CQRO^_ ∈ [Ω_N^CQRO^_^L^, Ω_N^CQRO^_^U^] for all x ∈ X, otherwise we called it an external NCq-ROF set.

**Definition 8 .**

The score functions under R-order of NCq-ROFNs

(11) $$\begin{array}{c} N_{i}^{CQRO}=\left\{\left(\left[{℧}_{N_{i}^{CQRO}}^{L},{℧}_{N_{i}^{CQRO}}^{U}\right],\left[\Omega_{N_{i}^{CQRO}}^{L},\Omega_{N_{i}^{CQRO}}^{U}\right]\right),\left(F_{N_{i}^{CQRO}},H_{N_{i}^{CQRO}}\right)\right\}, \end{array}$$

is define as

(12) $$\begin{array}{c} S\left(N_{i}^{CQRO}\right)=\frac{1{\left(-1\right)}^{2\overset{˘}{q}+1}}{2}\left[\frac{1}{4}\left[\begin{array}{c} \left(1+{\left({℧}_{N_{i}^{CQRO}}^{L}\right)}^{2\overset{˘}{q}}-{\left(\Omega_{N_{i}^{CQRO}}^{L}\right)}^{2\overset{˘}{q}}\right)+\\ \left(1+{\left({℧}_{N_{i}^{CQRO}}^{U}\right)}^{2\overset{˘}{q}}-{\left(\Omega_{N_{i}^{CQRO}}^{U}\right)}^{2\overset{˘}{q}}\right) \end{array}\right]+\left(F_{N_{i}^{CQRO}}^{2\overset{˘}{q}}-H_{N_{i}^{CQRO}}^{2\overset{˘}{q}}\right)\right], \end{array}$$

now for P-order, we get

(13) $$\begin{array}{c} S\left(N_{i}^{CQRO}\right)=\frac{1{\left(-1\right)}^{2\overset{˘}{q}+1}}{2}\left[\frac{1}{4}\left[\begin{array}{c} \left(1+{\left({℧}_{N_{i}^{CQRO}}^{L}\right)}^{2\overset{˘}{q}}-{\left(\Omega_{N_{i}^{CQRO}}^{L}\right)}^{2\overset{˘}{q}}\right)+\\ \left(1+{\left({℧}_{N_{i}^{CQRO}}^{U}\right)}^{2\overset{˘}{q}}-{\left(\Omega_{N_{i}^{CQRO}}^{U}\right)}^{2\overset{˘}{q}}\right) \end{array}\right]+\left(F_{N_{i}^{CQRO}}^{2\overset{˘}{q}}-H_{N_{i}^{CQRO}}^{2\overset{˘}{q}}\right)\right], \end{array}$$

and accuracy function is defined as

(14) $$\begin{array}{c} H\left(N_{i}^{CQRO}\right)=\frac{1{\left(-1\right)}^{2\overset{˘}{q}+1}}{2}\left[\frac{1}{2}\left[\begin{array}{c} \left({\left({℧}_{N_{i}^{CQRO}}^{L}\right)}^{2\overset{˘}{q}}+{\left({℧}_{N_{i}^{CQRO}}^{U}\right)}^{2\overset{˘}{q}}\right)+\\ \left({\left(\Omega_{N_{i}^{CQRO}}^{L}\right)}^{2\overset{˘}{q}}+{\left(\Omega_{N_{i}^{CQRO}}^{U}\right)}^{2\overset{˘}{q}}\right) \end{array}\right]+\left(F_{N_{i}^{CQRO}}^{2\overset{˘}{q}}+H_{N_{i}^{CQRO}}^{2\overset{˘}{q}}\right)\right], \end{array}$$

with the condition that

(15) $$\begin{array}{c} -1\leq S\left(N_{i}^{CQRO}\right)\leq 1,0\leq H\left(N_{i}^{CQRO}\right)\leq 1\text{.} \end{array}$$

**Definition 9 .**

The comparison rule for two NCq-ROFNs

(16) $$\begin{array}{c} N_{1}^{CQRO}=\left\{\left(\left[{℧}_{N_{1}^{CQRO}}^{L},{℧}_{N_{1}^{CQRO}}^{U}\right],\left[\Omega_{N_{1}^{CQRO}}^{L},\Omega_{N_{1}^{CQRO}}^{U}\right]\right),\left(F_{N_{1}^{CQRO}},H_{N_{1}^{CQRO}}\right)\right\}, \end{array}$$

and

(17) $$\begin{array}{c} N_{2}^{CQRO}=\left\{\left(\left[{℧}_{N_{2}^{CQRO}}^{L},{℧}_{N_{2}^{CQRO}}^{U}\right],\left[\Omega_{N_{2}^{CQRO}}^{L},\Omega_{N_{2}^{CQRO}}^{U}\right]\right),\left(F_{N_{2}^{CQRO}},H_{N_{2}^{CQRO}}\right)\right\}, \end{array}$$

are defined as

(1) If S(N_1_^CQRO^)≻S(N_2_^CQRO^), then N_1_^CQRO^≻N_2_^CQRO^. (2) If S(N_1_^CQRO^)=S(N_2_^CQRO^)(a)H(N_1_^CQRO^)≻H(N_2_^CQRO^), then N_1_^CQRO^≻N_2_^CQRO^(b)H(N_1_^CQRO^)=H(N_2_^CQRO^), then N_1_^CQRO^ ~ N_2_^CQRO^, where ″∼″ represent the “equivalent to.

**Example 1 .**

Assuming that N_1_^CQRO^={([−.7, −.2], [−.2, −.1]), (−.3, −.5)} andN_2_^CQRO^={([−.5, −.4], [−.4, −.3]), (−.2, −.7)} are two NCq-ROFNs, the score function under R-order *r* are defined as

(18) $$\begin{array}{c} S\left(N_{i}^{CQRO}\right)=\frac{1{\left(-1\right)}^{2\overset{˘}{q}+1}}{2}\left[\begin{array}{c} \frac{1}{4}\left[\begin{array}{c} \left(1+{\left({℧}_{N_{i}^{CQRO}}^{L}\right)}^{2\overset{˘}{q}}-{\left(\Omega_{N_{i}^{CQRO}}^{L}\right)}^{2\overset{˘}{q}}\right)+\\ \left(1+{\left({℧}_{N_{i}^{CQRO}}^{U}\right)}^{2\overset{˘}{q}}-{\left(\Omega_{N_{i}^{CQRO}}^{U}\right)}^{2\overset{˘}{q}}\right) \end{array}\right]\\ +\left(F_{N_{i}^{CQRO}}^{2\overset{˘}{q}}-H_{N_{i}^{CQRO}}^{2\overset{˘}{q}}\right) \end{array}\right],\\ S\left(N_{1}^{CQRO}\right)=\frac{1{\left(-1\right)}^{2\overset{˘}{q}+1}}{2}\left[\begin{array}{c} \frac{1}{4}\left[\begin{array}{c} \left(1+{\left(-.7\right)}^{2\overset{˘}{q}}-{\left(-.2\right)}^{2\overset{˘}{q}}\right)+\\ \left(1+{\left(-.2\right)}^{2\overset{˘}{q}}-{\left(-.1\right)}^{2\overset{˘}{q}}\right) \end{array}\right]\\ +\left({\left(-.3\right)}^{2\overset{˘}{q}}-{\left(-.5\right)}^{2\overset{˘}{q}}\right) \end{array}\right],\\ \begin{array}{cc} S\left(N_{1}^{CQRO}\right) & =\frac{1{\left(-1\right)}^{2\left(3\right)+1}}{2}\left[\begin{array}{c} \frac{1}{4}\left[\begin{array}{c} \left(1+{\left(-.7\right)}^{2\left(3\right)}-{\left(-.2\right)}^{2\left(3\right)}\right)+\\ \left(1+{\left(-.2\right)}^{2\left(3\right)}-{\left(-.1\right)}^{2\left(3\right)}\right) \end{array}\right]\\ +\left({\left(-.3\right)}^{2\left(3\right)}-{\left(-.5\right)}^{2\left(3\right)}\right) \end{array}\right],\\ S\left(N_{1}^{CQRO}\right) & =\frac{1{\left(-1\right)}^{7}}{2}\left[\begin{array}{c} \frac{1}{4}\left[\begin{array}{c} \left(1+{\left(-.7\right)}^{6}-{\left(-.2\right)}^{6}\right)+\\ \left(1+{\left(-.2\right)}^{6}-{\left(-.1\right)}^{6}\right) \end{array}\right]\\ +\left({\left(-.3\right)}^{6}-{\left(-.5\right)}^{6}\right) \end{array}\right],\\ S\left(N_{1}^{CQRO}\right) & =\frac{-1}{2}\left[\begin{array}{c} \frac{1}{4}\left[\left(1.117585\right)+\left(1.000063\right)\right]\\ +\left(\left(0.000729\right)-\left(0.15625\right)\right) \end{array}\right],\\ S\left(N_{1}^{CQRO}\right) & =\frac{-1}{2}\left[\begin{array}{c} \frac{1}{4}\left[2.117648\right]\\ +\left(-.155521\right) \end{array}\right],\\ S\left(N_{1}^{CQRO}\right) & =\frac{-1}{2}\left[0.529412-.155521\right],\\ S\left(N_{1}^{CQRO}\right) & =\frac{-1}{2}\left[0.3744202\right],\\ S\left(N_{1}^{CQRO}\right) & =-.1872101. \end{array} \end{array}$$

For

(19) $$\begin{array}{c} S\left(N_{2}^{CQRO}\right).S\left(N_{i}^{CQRO}\right)=\frac{1{\left(-1\right)}^{2\overset{˘}{q}+1}}{2}\left[\begin{array}{c} \frac{1}{4}\left[\begin{array}{c} \left(1+{\left({℧}_{N_{i}^{CQRO}}^{L}\right)}^{2\overset{˘}{q}}-{\left(\Omega_{N_{i}^{CQRO}}^{L}\right)}^{2\overset{˘}{q}}\right)+\\ \left(1+{\left({℧}_{N_{i}^{CQRO}}^{U}\right)}^{2\overset{˘}{q}}-{\left(\Omega_{N_{i}^{CQRO}}^{U}\right)}^{2\overset{˘}{q}}\right) \end{array}\right]\\ +\left(F_{N_{i}^{CQRO}}^{2\overset{˘}{q}}-H_{N_{i}^{CQRO}}^{2\overset{˘}{q}}\right) \end{array}\right],\\ S\left(N_{2}^{CQRO}\right)=\frac{1{\left(-1\right)}^{2\overset{˘}{q}+1}}{2}\left[\begin{array}{c} \frac{1}{4}\left[\begin{array}{c} \left(1+{\left(-.5\right)}^{2\overset{˘}{q}}-{\left(-.4\right)}^{2\overset{˘}{q}}\right)+\\ \left(1+{\left(-.4\right)}^{2\overset{˘}{q}}-{\left(-.3\right)}^{2\overset{˘}{q}}\right) \end{array}\right]\\ +\left({\left(-.2\right)}^{2\overset{˘}{q}}-{\left(-.7\right)}^{2\overset{˘}{q}}\right) \end{array}\right], \end{array}$$

where *q* = 3, then we get

(20) $$\begin{array}{c} S\left(N_{2}^{CQRO}\right)=\frac{1{\left(-1\right)}^{2\left(3\right)+1}}{2}\left[\begin{array}{c} \frac{1}{4}\left[\begin{array}{c} \left(1+{\left(-.5\right)}^{2\left(3\right)}-{\left(-.4\right)}^{2\left(3\right)}\right)+\\ \left(1+{\left(-.4\right)}^{2\left(3\right)}-{\left(-.3\right)}^{2\left(3\right)}\right) \end{array}\right]\\ +\left({\left(-.2\right)}^{2\left(3\right)}-{\left(-.7\right)}^{2\left(3\right)}\right) \end{array}\right],S\left(N_{2}^{CQRO}\right)=\frac{1{\left(-1\right)}^{7}}{2}\left[\begin{array}{c} \frac{1}{4}\left[\begin{array}{c} \left(1+{\left(-.5\right)}^{6}-{\left(-.4\right)}^{6}\right)+\\ \left(1+{\left(-.4\right)}^{6}-{\left(-.3\right)}^{6}\right) \end{array}\right]\\ +\left({\left(-.2\right)}^{6}-{\left(-.7\right)}^{6}\right) \end{array}\right],\\ \begin{array}{cc} S\left(N_{2}^{CQRO}\right) & =\frac{-1}{2}\left[\begin{array}{c} \frac{1}{4}\left[\left(1.011529\right)+\left(1.003367\right)\right]\\ +\left(\left(0.000064\right)-\left(0.117649\right)\right) \end{array}\right],\\ S\left(N_{2}^{CQRO}\right) & =\frac{-1}{2}\left[\begin{array}{c} \frac{1}{4}\left[2.014896\right]\\ +\left(-0/117585\right) \end{array}\right],\\ S\left(N_{2}^{CQRO}\right) & =\frac{-1}{2}\left[0.503724-0117585\right],\\ S\left(N_{2}^{CQRO}\right) & =\frac{-1}{2}\left[0.386139\right],\\ S\left(N_{2}^{CQRO}\right) & =-.1930696. \end{array} \end{array}$$

Now,

(21) $$\begin{array}{c} -.1872101≻-.1930696\\ S\left(N_{1}^{CQRO}\right)≻S\left(N_{2}^{CQRO}\right)\\ N_{1}^{CQRO}≻N_{2}^{CQRO} \end{array}$$

**Definition 10 .**

Considering the collection of NCq-ROFS to be N_*λ*_(*λ*=1,2,…n), j ≥ 0, k ≥ 0, if

(22) $$\begin{array}{c} NCq-ROFHM^{j,k}\left(N_{1},N_{2},\ldots ,N_{n}\right)={\left(\frac{2}{n\left(n+1\right)}\overset{n}{\underset{\lambda =1}{\sum }}\overset{n}{\underset{s=1}{\sum }}N_{\lambda }^{j}N_{s}^{j}\right)}^{1/j+k}. \end{array}$$

It is then referred to as an NCq-ROFHM operator.

**Theorem 1 .**

Assuming that j ≥ 0, k ≥ 0 and j+k ≥ 0, N_*λ*_=(Γ_N_*λ*__, Ϝ_N_*λ*__)(*λ*=1,2,…n) are a set of NCq-ROFNs, the results of solving equation (22) are also NCq-ROFSs.

(23) $$\begin{array}{c} NCq-ROFHM\left(\lambda_{1},\lambda_{2},\ldots \lambda_{n}\right)=\left\{\begin{array}{c} \left(\begin{array}{c} \left(\begin{array}{c} {\left(-1\right)}^{2\overset{˘}{q}+1}{\left[{\left({\left.1-{\left({℧}_{N_{\lambda }}^{L}\right)}^{j}{\left({℧}_{N_{S}}^{L}\right)}^{k}\right)}^{2\overset{˘}{q}}\right)}^{2/n\left(n+1\right)}\right]}^{1/2\overset{˘}{q}\left(j+k\right)},\\ {\left(-1\right)}^{2\overset{˘}{q}+1}{\left[{\left({\left.1-{\left({℧}_{N_{\lambda }}^{U}\right)}^{j}{\left({℧}_{N_{S}}^{U}\right)}^{k}\right)}^{2\overset{˘}{q}}\right)}^{2/n\left(n+1\right)}\right]}^{1/2\overset{˘}{q}\left(j+k\right)} \end{array}\right),\\ \left(\begin{array}{c} {\left(-1\right)}^{2\overset{˘}{q}+1}{\left(1-{\left(1-\Pi_{\lambda =1}^{n}\Pi_{s=1}^{n}{\left({1-{\left(\Omega_{N_{\lambda }}^{L}\right)}^{2\overset{˘}{q}}{\left(\right)}^{j}\left(1-{\left(\Omega_{Ns}^{L}\right)}^{2\overset{˘}{q}}\right)}^{k}\right)}^{2/n\left(n+1\right)}\right)}^{1/j+k}\right)}^{1/2q},\\ {\left(-1\right)}^{2\overset{˘}{q}+1}{\left(1-{\left(1-\Pi_{\lambda =1}^{n}\Pi_{s=1}^{n}{\left({1-{\left(\Omega_{N_{\lambda }}^{U}\right)}^{2\overset{˘}{q}}{\left(\right)}^{j}\left(1-{\left(\Omega_{Ns}^{U}\right)}^{2\overset{˘}{q}}\right)}^{k}\right)}^{2/n\left(n+1\right)}\right)}^{1/j+k}\right)}^{1/2q} \end{array}\right) \end{array}\right)\text{,}\\ \left(\begin{array}{c} {\left(-1\right)}^{2\overset{˘}{q}+1}{\left[{\left({\left.1-{\left({℧}_{N_{\lambda }}\right)}^{j}{\left({℧}_{N_{S}}\right)}^{k}\right)}^{2\overset{˘}{q}}\right)}^{2/n\left(n+1\right)}\right]}^{1/2\overset{˘}{q}\left(j+k\right)},\\ {\left(-1\right)}^{2\overset{˘}{q}+1}{\left(1-{\left(1-\Pi_{\lambda =1}^{n}\Pi_{s=1}^{n}{\left({1-{\left(\Omega_{N_{\lambda }}\right)}^{2\overset{˘}{q}}\left(1-{\left(\Omega_{Ns}\right)}^{2\overset{˘}{q}}\right)}^{k}\right)}^{2/n\left(n+1\right)}\right)}^{1/j+k}\right)}^{1/2q} \end{array}\right)\text{,} \end{array}\right\}. \end{array}$$

(Idempotency) Consider N_*λ*_=N(A_N_*λ*__, B_N_S__)(*λ*=1,2,…n) be a collection of NCq-ROFNS, if allN_*λ*_ are identical, that is N_*λ*_=N=(A_N_*λ*__, B_N_S__) for all *λ*, then NCq-ROFHM^j,k ^(N_1_, N_2_, N_n_)=N.

Proof As, N_*λ*_=N, ∀*λ* we have

(24) $$\begin{array}{c} NCq-ROFHM^{j,k}\left(N_{1},N_{2},..,N_{n}\right)={\left(\frac{2}{n\left(n+1\right)}\overset{n}{\underset{\lambda =1}{\sum }}\overset{n}{\underset{s=\lambda }{\sum }}N_{\lambda }^{j}N_{s}^{k}\right)}^{1/j+k}={\left(N^{j+k}\right)}^{1/j+k}=N\text{.} \end{array}$$

(Monotonicity):Let *α*_*λ*_, *β*_*λ*_(*λ*=1,2, ..n) represent the two NCq-ROFN families, if *α*_*λ*_ ≤ *β*_*λ*_∀ *λ*=1,2,…, n then

(25) $$\begin{array}{c} NCq-ROFHM^{j,k}\left(\alpha_{1},\alpha_{2},\ldots ,\alpha_{n}\right)\leq NCq-ROFHM^{j,k}\left(\beta_{1},\beta_{2},\ldots \beta_{n}\right)\text{.} \end{array}$$

**Proof**

Since, *α*_*λ*_ ≤ *β*_*λ*_ and *α*_s_ ≤ *β*_s_ for *λ*=1,2, ..n and s=i, i+1,…, n, we have

(26) $$\begin{array}{c} \alpha_{\lambda }^{j}\alpha_{s}^{k}\leq \beta_{\lambda }^{j}\beta_{s}^{k}. \end{array}$$

then

(27) $$\begin{array}{c} \frac{2}{n\left(n+1\right)}\overset{n}{\underset{\lambda =1}{\sum }}\overset{n}{\underset{s=\lambda }{\sum }}{\alpha_{\lambda }^{j}\alpha }_{s}^{k}\leq \frac{2}{n\left(n+1\right)}\overset{n}{\underset{\lambda =1}{\sum }}\overset{n}{\underset{s=\lambda }{\sum }}\beta_{\lambda }^{j}\beta_{s}^{k}\text{,} \end{array}$$

so,

(28) $$\begin{array}{c} {\left(\frac{2}{n\left(n+1\right)}\overset{n}{\underset{\lambda =1}{\sum }}\overset{n}{\underset{s=\lambda }{\sum }}\alpha_{\lambda }^{j}\alpha_{s}^{k}\right)}^{1/j+k}\leq {\left(\frac{2}{n\left(n+1\right)}\overset{n}{\underset{\lambda =1}{\sum }}\overset{n}{\underset{s=\lambda }{\sum }}\beta_{\lambda }^{j}\beta_{s}^{k}\right)}^{1/j+k}. \end{array}$$

And,

(29) $$\begin{array}{c} NCq-ROFHM^{j,k}\left(\alpha_{1},\alpha_{2},\ldots ,\alpha_{n}\right)\leq NCq-ROFHM^{j,k}\left(\beta_{1},\beta_{2},\ldots ,\beta_{n}\right)\text{.} \end{array}$$

(Boundedness). Between the max and min operators is the NCq-ROFHM operator.

(30) $$\begin{array}{c} \min\;\left(N_{1},N_{2},\ldots ,N_{n}\right)\leq NCq-ROFHM^{j,k}\left(N_{1},N_{2},\ldots ,N_{n}\right)\leq \max\;\left(N_{1},N_{2},\ldots ,N_{n}\right)\text{.} \end{array}$$

**Proof**

Let c=min(N_1_, N_2_,…, N_n_), d=max(N_1_, N_2_,…, N_n_).

Using the aforementioned theorem, we obtain

(31) $$\begin{array}{c} NCq-ROFHM^{j,k}\left(c,c,\ldots c\right)\leq NqQ-ROFHM^{j,k}\left(N_{1},N_{2},\ldots ,N_{n}\right)\leq NCq-ROFHM^{j,k}\left(d,d,\ldots ,d\right)\text{.} \end{array}$$

And,

(32) $$\begin{array}{c} \min\;\left(N_{1},N_{2},\ldots ,N_{n}\right)\leq NCq-ROFHM^{j,k}\left(N_{1},N_{2},\ldots ,N_{n}\right)\leq \max\;\left(N_{1},N_{2},\ldots ,N_{n}\right)\text{.} \end{array}$$

**Case 1 .**

The assertion that the recommended NCq-ROFHM operator transforms into the NCq-ROF basic HM operator if *j* = *k*=(1/2).

(33) $$\begin{array}{c} NCq-ROFHM^{1/21/2}\left(N_{1},N_{2},\ldots ,N_{n}\right)=\begin{array}{c} \left(\begin{array}{c} \left[\begin{array}{c} {\left(-1\right)}^{2\overset{˘}{q}+1}{\left(1-\Pi_{\lambda =1}^{n}\Pi_{s=\lambda }^{n}{\left(1-\sqrt{{\left({℧}_{N_{\lambda }}^{L}{℧}_{N_{S}}^{L}\right)}^{2\overset{˘}{q}}}\right)}^{2/n\left(n+1\right)}\right)}^{1/2\overset{˘}{q}},\\ {\left(-1\right)}^{2\overset{˘}{q}+1}{\left(1-\Pi_{\lambda =1}^{n}\Pi_{s=\lambda }^{n}{\left(1-\sqrt{{\left({℧}_{N_{\lambda }}^{U}{℧}_{N_{S}}^{U}\right)}^{2\overset{˘}{q}}}\right)}^{2/n\left(n+1\right)}\right)}^{1/2\overset{˘}{q}} \end{array}\right],\\ \left[\begin{array}{c} {\left(-1\right)}^{2\overset{˘}{q}+1}\left(\Pi_{\lambda =1}^{n}\Pi_{s=\lambda }^{n}{\left(1-\sqrt{\left(\left(1-{\left(\Omega_{N_{\lambda }}^{L}\right)}^{2\overset{˘}{q}}\right)\left(1-{\left(\Omega_{N_{\lambda }}^{L}\right)}^{2\overset{˘}{q}}\right)\right)}\right)}^{2/n\left(n+1\right)*1/2\overset{˘}{q}}\right),\\ {\left(-1\right)}^{2\overset{˘}{q}+1}\left(\Pi_{\lambda =1}^{n}\Pi_{s=\lambda }^{n}{\left(1-\sqrt{\left(\left(1-{\left(\Omega_{N_{\lambda }}^{U}\right)}^{2\overset{˘}{q}}\right)\left(1-{\left(\Omega_{N_{\lambda }}^{U}\right)}^{2\overset{˘}{q}}\right)\right)}\right)}^{2/n\left(n+1\right)*1/2\overset{˘}{q}}\right) \end{array}\right], \end{array}\right),\\ \left(\left(\begin{array}{c} {\left(-1\right)}^{2\overset{˘}{q}+1}{\left(1-\Pi_{\lambda =1}^{n}\Pi_{s=\lambda }^{n}{\left(1-\sqrt{{\left({℧}_{N_{\lambda }}{℧}_{N_{S}}\right)}^{2\overset{˘}{q}}}\right)}^{2/n\left(n+1\right)}\right)}^{1/2\overset{˘}{q}},\\ {\left(-1\right)}^{2\overset{˘}{q}+1}\left(\Pi_{\lambda =1}^{n}\Pi_{s=\lambda }^{n}{\left(1-\sqrt{\left(\left(1-{\left(\Omega_{N_{\lambda }}\right)}^{2\overset{˘}{q}}\right)\left(1-{\left(\Omega_{N_{s}}\right)}^{2\overset{˘}{q}}\right)\right)}\right)}^{2/n\left(n+1\right)*1/2\overset{˘}{q}}\right) \end{array}\right)\right). \end{array} \end{array}$$

**Case 2 .**

If j=k=1 then (14) change into

(34) $$\begin{array}{c} NCQ-ROFHM^{1,1}\left(N_{1},N_{2},\ldots ,N_{n}\right)\\ =\left\{\begin{array}{c} \left(\begin{array}{c} \left[\begin{array}{c} {\left(-1\right)}^{2\overset{˘}{q}+1}{\left(1-\Pi_{\lambda =1}^{n}\Pi_{s=\lambda }^{n}{\left(1-{\left({℧}_{N_{\lambda }}^{L}{℧}_{N_{S}}^{L}\right)}^{2\overset{˘}{q}}\right)}^{2/n\left(n+1\right)}\right)}^{1/4\overset{˘}{q}},\\ {\left(-1\right)}^{2\overset{˘}{q}+1}{\left(1-\Pi_{\lambda =1}^{n}\Pi_{s=\lambda }^{n}{\left(1-{\left({℧}_{N_{\lambda }}^{U}{℧}_{N_{S}}^{U}\right)}^{2\overset{˘}{q}}\right)}^{2/n\left(n+1\right)}\right)}^{1/4\overset{˘}{q}} \end{array}\right],\\ {\left(-1\right)}^{2\overset{˘}{q}+1}{\left(1-{\left(1-\Pi_{\lambda =1}^{n}\Pi_{s=\lambda }^{n}{\left(1-1-{\left(\Omega_{N_{\lambda }}^{L}\right)}^{2\overset{˘}{q}}\left(1-{\left(\Omega_{N_{s}}^{L}\right)}^{2\overset{˘}{q}}\right)\right)}^{2/n\left(n+1\right)}\right)}^{1/2}\right)}^{1/2\overset{˘}{q}}\\ {\left(-1\right)}^{2\overset{˘}{q}+1}{\left(1-{\left(1-\Pi_{\lambda =1}^{n}\Pi_{s=\lambda }^{n}{\left(1-1-{\left(\Omega_{N_{\lambda }}^{U}\right)}^{2\overset{˘}{q}}\left(1-{\left(\Omega_{N_{s}}^{U}\right)}^{2\overset{˘}{q}}\right)\right)}^{2/n\left(n+1\right)}\right)}^{1/2}\right)}^{1/2\overset{˘}{q}} \end{array}\right)\text{,}\\ \left(\begin{array}{c} {\left(-1\right)}^{2\overset{˘}{q}+1}{\left(1-\Pi_{\lambda =1}^{n}\Pi_{s=\lambda }^{n}{\left(1-{\left({℧}_{N_{\lambda }}{℧}_{N_{S}}\right)}^{2\overset{˘}{q}}\right)}^{2/n\left(n+1\right)}\right)}^{1/2\overset{˘}{q}},\\ {\left(-1\right)}^{2\overset{˘}{q}+1}{\left(1-{\left(1-\Pi_{\lambda =1}^{n}\Pi_{s=\lambda }^{n}{\left(1-\left(1-{\left(\Omega_{N_{\lambda }}\right)}^{2\overset{˘}{q}}\right)\left(1-{\left(\Omega_{N_{s}}\right)}^{2\overset{˘}{q}}\right)\right)}^{2/n\left(n+1\right)}\right)}^{1/2}\right)}^{1/2\overset{˘}{q}} \end{array}\right) \end{array}\right\}. \end{array}$$

This means that it is also referred to as the N-cubic Q-rung orthopair fuzzy generalized interconnected square mean.

**Case 3 .**

If *j*⟶0, (34) is reduced to

(35) $$\begin{array}{c} \lim_{j⟶0}\;NCQ-ROFHM^{j,k}\left(N_{1},N_{2},\ldots ,N_{n}\right)={\left(\frac{1}{n}\overset{n}{\underset{\lambda =1}{\sum }}N_{\lambda }^{j}\right)}^{1/j}\\ =\left\{\begin{array}{c} \left(\begin{array}{c} \left[\begin{array}{c} {\left(-1\right)}^{2\overset{˘}{q}+1}{\left(1-\Pi_{\lambda =1}^{n}\left({\left(1-{\left({\left({℧}_{N_{\lambda }}^{L}\right)}^{k}\right)}^{2\overset{˘}{q}}\right)}^{1/n}\right)\right)}^{1/j+k},\\ {\left(-1\right)}^{2\overset{˘}{q}+1}{\left(1-\Pi_{\lambda =1}^{n}\left({\left(1-{\left({\left({℧}_{N_{\lambda }}^{U}\right)}^{k}\right)}^{2\overset{˘}{q}}\right)}^{1/n}\right)\right)}^{1/j+k} \end{array}\right],\\ \left[\begin{array}{c} {\left(-1\right)}^{2\overset{˘}{q}+1}{\left(1-{\left(1-\Pi_{\lambda =1}^{n}{\left(1-\left(1-{\left({\left(\Omega_{N_{\lambda }}^{L}\right)}^{2\overset{˘}{q}}\right)}^{k}\right)\right)}^{1/n}\right)}^{1/k}\right)}^{1/2\overset{˘}{q}},\\ {\left(-1\right)}^{2\overset{˘}{q}+1}{\left(1-{\left(1-\Pi_{\lambda =1}^{n}{\left(1-\left(1-{\left({\left(\Omega_{N_{\lambda }}^{U}\right)}^{2\overset{˘}{q}}\right)}^{k}\right)\right)}^{1/n}\right)}^{1/k}\right)}^{1/2\overset{˘}{q}} \end{array}\right] \end{array}\right),\\ \left(\begin{array}{c} {\left(-1\right)}^{2\overset{˘}{q}+1}{\left(1-\Pi_{\lambda =1}^{n}\left({\left(1-{\left({\left({℧}_{N_{\lambda }}\right)}^{k}\right)}^{2\overset{˘}{q}}\right)}^{1/n}\right)\right)}^{1/j+k},\\ {\left(-1\right)}^{2\overset{˘}{q}+1}{\left(1-{\left(1-\Pi_{\lambda =1}^{n}{\left(1-{\left(1-\left({\left(\Omega_{N_{\lambda }}\right)}^{2\overset{˘}{q}}\right)\right)}^{k}\right)}^{1/n}\right)}^{1/k}\right)}^{1/2\overset{˘}{q}} \end{array}\right) \end{array}\right\}. \end{array}$$

It is sometimes referred to as the N-cubic q-rung s fuzzy generalized mean.

**Case 4 .**

If *j*=1 and *k*⟶0, (27) becomes an N-cubic q-rung orthopair fuzzy average mean.

(36) $$\begin{array}{c} \lim_{k⟶0}NCQ-ROFHM^{j,k}\left(N_{1},N_{2},\ldots ,N_{n}\right)\\ =\left(\frac{1}{n}{⊗}_{\lambda =1}^{n}N_{\lambda }\right)\\ =\left\{\begin{array}{c} \left(\begin{array}{c} \left[\begin{array}{c} {\left(-1\right)}^{2\overset{˘}{q}+1}{\left(1-{⊗}_{\lambda =1}^{n}{\left(1-{\left({℧}_{N_{\lambda }}^{L}\right)}^{2\overset{˘}{q}}\right)}^{2/n}\right)}^{1/2q},\\ {\left(-1\right)}^{2\overset{˘}{q}+1}{\left(1-{⊗}_{\lambda =1}^{n}{\left(1-{\left({℧}_{N_{\lambda }}^{U}\right)}^{2\overset{˘}{q}}\right)}^{2/n}\right)}^{1/2q} \end{array}\right],\\ \left[\begin{array}{c} {\left(-1\right)}^{2\overset{˘}{q}+1}{\left(1-\left(1-{⊗}_{\lambda =1}^{n}{\left(1-\left(1-{\left(\Omega_{N_{\lambda }}^{L}\right)}^{2\overset{˘}{q}}\right)\right)}^{1/n}\right)\right)}^{1/2q},\\ {\left(-1\right)}^{2\overset{˘}{q}+1}{\left(1-\left(1-{⊗}_{\lambda =1}^{n}{\left(1-\left(1-{\left(\Omega_{N_{\lambda }}^{U}\right)}^{2\overset{˘}{q}}\right)\right)}^{1/n}\right)\right)}^{1/2q} \end{array}\right] \end{array}\right)\text{,}\\ \left(\begin{array}{c} {\left(-1\right)}^{2\overset{˘}{q}+1}{\left(1-{⊗}_{\lambda =1}^{n}{\left(1-{\left({℧}_{N_{\lambda }}\right)}^{2\overset{˘}{q}}\right)}^{1/n}\right)}^{\frac{1}{2\overset{˘}{q}}},\\ {\left(-1\right)}^{2\overset{˘}{q}+1}{\left(1-\left(1-{⊗}_{\lambda =1}^{n}{\left(1-\left(1-{\left(\Omega_{N_{\lambda }}\right)}^{2\overset{˘}{q}}\right)\right)}^{1/n}\right)\right)}^{1/2q} \end{array}\right) \end{array}\right\}. \end{array}$$

**Case 5 .**

If *j*⟶0, *k*⟶0, then the existing NCq-ROFHM change into

(37) $$\begin{array}{c} \lim_{j⟶0}NqQ-ROFHM^{j,0}\left(N_{1},N_{2},\ldots ,N_{n}\right)=\lim_{k⟶0}{\left(\frac{1}{n}{⊗}_{\lambda =1}^{n}N_{\lambda }^{j}\right)}^{1/k}={⊗}_{\lambda =1}^{n}{\left(N_{\lambda }\right)}^{1/n}\text{.} \end{array}$$

Note that we can get a variety of orthopair fuzzy sets by varying the value of the parameter *q*. As an illustration, the N-cubic Pythagorean fuzzy set is renovated by NCq-ROFHM if *j* = 1 and *k* = 1. In MADM situations, different characteristics typically have significant advantages. Thus, it appears that the NCq-ROFHM operator is indifferent with this characteristic. The weighted version of the NCq-ROFHM operator is defined as follows to address this issue:

**Definition 11 .**

In this case, *N*_*λ*_=(*A*_*N*_*λ*__, *B*_*N*_*λ*__)(*λ*=1,2,…, *n*) be the NCq-ROFN family, the weight vector of NCq-ROFNs is indicated by *j* ≥ 0, *k* ≥ 0, *j*+*k* ≥ 0, and *w*=(*w*_1_, *w*_2_,…, *w*_*n*_) for all *w*_*λ*_ ∈ [0,1] and ∑_*λ*=1_^*n*^*w*=1.Then NCq-ROFWHM: [−1,0]^*n*^⟶[−1,0] such that

(38) $$\begin{array}{c} NCq-ROFWHM_{w}^{j,k}\left(N_{1},N_{2},\ldots ,N_{n}\right)={\left(\frac{2}{n\left(n+1\right)}\overset{n}{\underset{\lambda =1}{\sum }}\overset{n}{\underset{s=1}{\sum }}{\left(w_{\lambda }N_{\lambda }\right)}^{j}{\left(w_{s}N_{s}\right)}^{k}\right)}^{1/j+k}. \end{array}$$

**Theorem 2 .**

Let *N*_*λ*_=(*A*_*N*_*λ*__, *B*_*N*_*λ*__)(*λ*=1,2,…, *n*) be the collection of NCq-ROFNs, j ≥ 0, *k* ≥ 0 and *j*+*k* ≥ 0, and *w*=(*w*_1_, *w*_2_,…, *w*_*n*_) represents the weight vector of NCq-ROFNs, *w*_*λ*_ ∈ [0,1] and ∑_*λ*=1_^*n*^*w*=1. Then, NCq-ROFNs are also included in the resulting equation (38) as

(39) $$\begin{array}{c} NCq-ROFWHM_{w}^{j,k}\left(N_{1},N_{2},\ldots ,N_{n}\right)=\left\{\begin{array}{c} \left[\begin{array}{c} \left[\begin{array}{c} {\left(-1\right)}^{2\overset{˘}{q}+1}{\left(1-\Pi_{\lambda =1}^{n}\Pi_{s=\lambda }^{n}{\left(1-{\left({℧}_{N_{\lambda }}^{L}\right)}^{2\overset{˘}{q}}\right)}^{2/n\left(n+1\right)}\right)}^{1/2\overset{˘}{q}\left(j+k\right)},\\ {\left(-1\right)}^{2\overset{˘}{q}+1}{\left(1-\Pi_{\lambda =1}^{n}\Pi_{s=\lambda }^{n}{\left(1-{\left({℧}_{N_{\lambda }}^{U}\right)}^{2\overset{˘}{q}}\right)}^{2/n\left(n+1\right)}\right)}^{1/2\overset{˘}{q}\left(j+k\right)} \end{array}\right],\\ \left[\begin{array}{c} {\left(-1\right)}^{2\overset{˘}{q}+1}{\left(1-{\left(1-\Pi_{\lambda =1}^{n}\Pi_{s=\lambda }^{n}{\left(\Omega_{N_{\lambda }}^{L}\right)}^{4q/n\left(n+1\right)}\right)}^{1/j+k}\right)}^{1/2\overset{˘}{q}},\\ {\left(-1\right)}^{2\overset{˘}{q}+1}{\left(1-{\left(1-\Pi_{\lambda =1}^{n}\Pi_{s=\lambda }^{n}{\left(\Omega_{N_{\lambda }}^{U}\right)}^{4q/n\left(n+1\right)}\right)}^{1/j+k}\right)}^{1/2\overset{˘}{q}} \end{array}\right] \end{array}\right]\text{,}\\ \left(\begin{array}{c} \left({\left(-1\right)}^{2\overset{˘}{q}+1}{\left(1-\Pi_{\lambda =1}^{n}\Pi_{s=\lambda }^{n}{\left(1-{\left({℧}_{N_{\lambda }}\right)}^{2\overset{˘}{q}}\right)}^{2/n\left(n+1\right)}\right)}^{1/2\overset{˘}{q}\left(j+k\right)}\right),\\ {\left(-1\right)}^{2\overset{˘}{q}+1}{\left(1-{\left(1-\Pi_{\lambda =1}^{n}\Pi_{s=\lambda }^{n}{\left(\Omega_{N_{\lambda }}\right)}^{4q/n\left(n+1\right)}\right)}^{1/j+k}\right)}^{1/2\overset{˘}{q}} \end{array}\right) \end{array}\right\}. \end{array}$$

where

(40) $$\begin{array}{c} \left[{℧}_{\lambda }^{L},{℧}_{\lambda }^{U}\right]=\left[\begin{array}{c} {\left(-1\right)}^{2\overset{˘}{q}+1}\left({\left(1-{\left(1-{\left({℧}_{\lambda }^{L}\right)}^{2\overset{˘}{q}}\right)}^{w_{\lambda }}\right)}^{j/2\overset{˘}{q}}{\left(1-{\left(1-{\left({℧}_{s}^{L}\right)}^{2\overset{˘}{q}}\right)}^{w_{s}}\right)}^{k/2\overset{˘}{q}}\right)\text{,}\\ {\left(-1\right)}^{2\overset{˘}{q}+1}\left({\left(1-{\left(1-{\left({℧}_{\lambda }^{U}\right)}^{2\overset{˘}{q}}\right)}^{w_{\lambda }}\right)}^{j/2\overset{˘}{q}}{\left(1-{\left(1-{\left({℧}_{s}^{U}\right)}^{2\overset{˘}{q}}\right)}^{w_{s}}\right)}^{k/2\overset{˘}{q}}\right) \end{array}\right]\text{,}\\ \left[\Omega_{\lambda }^{L},\Omega_{\lambda }^{U}\right]=\left[\begin{array}{c} {\left(-1\right)}^{2\overset{˘}{q}+1}{\left(1-{\left(1-{\left(\Omega_{\lambda }^{L}\right)}^{2\overset{˘}{q}w_{\lambda }}\right)}^{j}{\left(1-{\left(\Omega_{s}^{L}\right)}^{2\overset{˘}{q}w_{s}}\right)}^{k}\right)}^{1/2\overset{˘}{q}}\text{,}\\ {\left(-1\right)}^{2\overset{˘}{q}+1}{\left(1-{\left(1-{\left(\Omega_{\lambda }^{U}\right)}^{2\overset{˘}{q}w_{\lambda }}\right)}^{j}{\left(1-{\left(\Omega_{s}^{U}\right)}^{2\overset{˘}{q}w_{s}}\right)}^{k}\right)}^{1/2\overset{˘}{q}} \end{array}\right]\text{,}\\ {℧}_{\lambda }={\left(-1\right)}^{2\overset{˘}{q}+1}\left({\left(1-{\left(1-{\left({℧}_{\lambda }\right)}^{2\overset{˘}{q}}\right)}^{w_{\lambda }}\right)}^{j/2\overset{˘}{q}}{\left(1-{\left(1-{\left({℧}_{s}\right)}^{2\overset{˘}{q}}\right)}^{w_{s}}\right)}^{k/2\overset{˘}{q}}\right)\text{,}\\ \Omega_{\lambda }={\left(-1\right)}^{2\overset{˘}{q}+1}{\left(1-{\left(1-{\left(\Omega_{\lambda }\right)}^{2\overset{˘}{q}w_{\lambda }}\right)}^{j}{\left(1-{\left(\Omega_{s}\right)}^{2\overset{˘}{q}w_{s}}\right)}^{k}\right)}^{1/2\overset{˘}{q}}. \end{array}$$

The relationship between the structure of the two attributes can be established through the HM operator. Each attribute is linked with other attributes of the HM operator. However, when it comes to decision-making issues, this condition is often not being met. To prevent the separation of characteristics we can use different partitions to solve decision-making problems because we remember the structure of attribute relationships. There is no link between attributes. When they are divided by two partitions, the same attributes present in partitions have a connection to each other. With the typical HM operator, the partitions do not solve these kinds of issues so we now provide the N-cubic q-rung orthopair fuzzy power Hamy mean operator with the ability to let us know the issue. The condition given above can be mathematically explained as: Let *N*_*λ*_=(*A*_*N*_*λ*__, *B*_*N*_*λ*__)(*λ*=1,2, ..n) be a collection of NCq-ROFNs, distributed into “*g*” different partitions F*F*_1_,*F*_2_,….,*F*_*g*_ with $F_{i}\cap F_{\tilde{ı}}$ and ∪_*i*=1_^*g*^*F*_*i*_={*N*_*i*_}*F*_*i*_={*N*_*i*1_, *N*_*i*2_,…*N*_*i*|*F*_*i*_|_}, where |*F*_*i*_| denotes the cardinality of partitions *F*_*i*_ and ∑_*i*=1_^*g*^|*F*_*i*_|=*n*. By using above information, NCQ-ROFPHM operator is defined as

**Definition 12 .**

Let *N*_*λ*_=(*A*_*N*_*λ*__, *B*_*N*_*λ*__)(*λ*=1,2, ..*n*) be a family of NCq-ROFNs,

*j* ≥ 0, *k* ≥ 0 and *j*+*k* ≥ 0. Then NCq-ROFPHM [−1,0]^*n*^⟶[−1,0] and

(41) $$\begin{array}{c} NCq-ROFPHM^{j,k}\left(N_{1},N_{2},\ldots ,N_{n}\right)=\frac{1}{g}\left(\overset{g}{\underset{i=1}{\sum }}{\left(\frac{2}{\left|F_{i}\right|\left(\left|F_{i}\right|+1\right)}\overset{\left|F_{i}\right|}{\underset{\lambda =1}{\sum }}\overset{\left|F_{i}\right|}{\underset{s=\lambda }{\sum }}{\left(N_{i\lambda }\right)}^{j}⊗{\left(N_{is}\right)}^{k}\right)}^{1/j+k}\right). \end{array}$$

**Theorem 3 .**

Let *N*_*λ*_=(*A*_*N*_*λ*__, *B*_*N*_*λ*__)(*λ*=1,2, ..*n*) be a family of NCq-ROFNs, *j* ≥ 0, *k* ≥ 0 and *j*+*k* ≥ 0, then equation (41) is used to generate a consequent equation that is likewise an NCq-ROFN, as shown by

(42) $$\begin{array}{c} NCq-ROFPHM^{j,k\;}\left(N_{1},N_{2},\ldots ,N_{n}\right)=\left\{\left(\begin{array}{c} \left(\begin{array}{c} \left[\begin{array}{c} {\left(-1\right)}^{2\overset{˘}{q}+1}{\left(1-\Pi_{i=1}^{g}{\left(1-{\left({\left(1-\left(1-{\left({℧}_{i}^{L}\right)}^{2\overset{˘}{q}}\right)\right)}^{2/\left|F_{i}\right|\left(\left|F_{i}\right|+1\right)}\right)}^{1/j+k}\right)}^{1/g}\right)}^{1/2\overset{˘}{q}},\\ {\left(-1\right)}^{2\overset{˘}{q}+1}{\left(1-\Pi_{i=1}^{g}{\left(1-{\left({\left(1-\left(1-{\left({℧}_{i}^{U}\right)}^{2\overset{˘}{q}}\right)\right)}^{2/\left|F_{i}\right|\left(\left|F_{i}\right|+1\right)}\right)}^{1/j+k}\right)}^{1/g}\right)}^{1/2\overset{˘}{q}} \end{array}\right],\\ \left[\begin{array}{c} {\left(-1\right)}^{2\overset{˘}{q}+1}\left(\Pi_{i=1}^{g}{\left(1-{\left(1-{\left(\Omega_{i}^{L}\right)}^{4q/\left|F_{i}\right|\left(\left|F_{i}\right|+1\right)}\right)}^{1/j+k}\right)}^{1/q*g}\right),\\ {\left(-1\right)}^{2\overset{˘}{q}+1}\left(\Pi_{i=1}^{g}{\left(1-{\left(1-{\left(\Omega_{i}^{L}\right)}^{4q/\left|F_{i}\right|\left(\left|F_{i}\right|+1\right)}\right)}^{1/j+k}\right)}^{1/q*g}\right) \end{array}\right] \end{array}\right)\text{,}\\ \left(\begin{array}{c} {\left(-1\right)}^{2\overset{˘}{q}+1}{\left(1-\Pi_{i=1}^{g}{\left(1-{\left(\left(1-{\left(1-{\left({℧}_{i}\right)}^{2\overset{˘}{q}}\right)}^{2/\left|F_{i}\right|\left(\left|F_{i}\right|+1\right)}\right)\right)}^{1/j+k}\right)}^{1/g}\right)}^{1/2\overset{˘}{q}},\\ {\left(-1\right)}^{2\overset{˘}{q}+1}\left(\Pi_{i=1}^{g}{\left(1-{\left(1-{\left(\Omega_{i}\right)}^{4q/\left|F_{i}\right|\left(\left|F_{i}\right|+1\right)}\right)}^{1/j+k}\right)}^{1/q*g}\right) \end{array}\right) \end{array}\right)\right\}, \end{array}$$

Where

(43) $$\begin{array}{c} {℧}_{i}^{L}={\left(-1\right)}^{2\overset{˘}{q}+1}{\left(1-\Pi_{\lambda =1}^{\left|Fi\right|}\Pi_{s=\lambda }^{\left|Fi\right|}\left(1-{\left(A_{N_{i\lambda }}^{j}B_{Ni_{s}}^{k}\right)}^{q}\right)\right)}^{1/\overset{˘}{q}}\text{,}\\ {℧}_{i}^{U}={\left(-1\right)}^{2\overset{˘}{q}+1}{\left(1-\Pi_{\lambda =1}^{\left|Fi\right|}\Pi_{s=\lambda }^{\left|Fi\right|}\left(1-{\left(A_{N_{i\lambda }}^{j}B_{Ni_{s}}^{k}\right)}^{q}\right)\right)}^{1/\overset{˘}{q}},\\ \Omega_{i}^{L}={\left(-1\right)}^{2\overset{˘}{q}+1}\left(\Pi_{\lambda =1}^{\left|Fi\right|}\Pi_{s=\lambda }^{\left|Fi\right|}{\left(1-{\left(1-B_{N_{i\lambda }}^{2\overset{˘}{q}}\right)}^{j}{\left(1-B_{N_{is}}^{2\overset{˘}{q}}\right)}^{k}\right)}^{1/2\overset{˘}{q}}\right)\text{,}\\ \Omega_{i}^{U}={\left(-1\right)}^{2\overset{˘}{q}+1}\left(\Pi_{\lambda =1}^{\left|Fi\right|}\Pi_{s=\lambda }^{\left|Fi\right|}{\left(1-{\left(1-B_{N_{i\lambda }}^{2\overset{˘}{q}}\right)}^{j}{\left(1-B_{N_{is}}^{2\overset{˘}{q}}\right)}^{k}\right)}^{1/2\overset{˘}{q}}\right),\\ {℧}_{i}={\left(-1\right)}^{2\overset{˘}{q}+1}{\left(1-\Pi_{\lambda =1}^{\left|Fi\right|}\Pi_{s=\lambda }^{\left|Fi\right|}\left(1-{\left(A_{N_{i\lambda }}^{j}B_{Ni_{s}}^{k}\right)}^{2\overset{˘}{q}}\right)\right)}^{1/2\overset{˘}{q}}\text{,}\\ \Omega_{i}={\left(-1\right)}^{2\overset{˘}{q}+1}\left(\Pi_{\lambda =1}^{\left|Fi\right|}\Pi_{s=\lambda }^{\left|Fi\right|}{\left(1-{\left(1-B_{N_{i\lambda }}^{2\overset{˘}{q}}\right)}^{j}{\left(1-B_{N_{is}}^{2\overset{˘}{q}}\right)}^{k}\right)}^{1/2\overset{˘}{q}}\right). \end{array}$$

**Theorem 4 .**

Let *j* ≥ 0, *k* ≥ 0 *j*+*k* ≥ 0,

(44) $$\begin{array}{c} N_{\lambda }=\left(A_{N_{\lambda }},B_{N_{\lambda }}\right)\left(\lambda =1,2,\ldots ,n\right). \end{array}$$

Be collection of NCq-ROFNs with *g* different subset *F*_*λ*_(*λ*=1,2,…, *n*). Consequently, the NCq-ROFPHM operators have the following characteristics.

(Idempotency) If all *N*_*λ*_ are same that is, *N*_*λ*_=*N*=(*A*_*N*_, *B*_*N*_)∀ *λ* then

(45) $$\begin{array}{c} NCq-ROFPHM^{j,k}\left(N_{1},N_{2},\ldots ,N_{n}\right)=N=\left(A_{N},B_{N}\right)\text{,} \end{array}$$

**Proof**

(46) $$\begin{array}{c} \begin{array}{c} NCq-ROFPHM^{j,k}\left(N_{1},N_{2},\ldots ,N_{n}\right)=\frac{1}{g}\left(\overset{g}{\underset{i=1}{\sum }}{\left(\frac{2}{\left|F_{i}\right|\left(\left|F_{i}\right|+1\right)}\overset{\left|F_{i}\right|}{\underset{\lambda =1}{\sum }}\overset{\left|F_{i}\right|}{\underset{s=\lambda }{\sum }}{\left(N_{i\lambda }\right)}^{j}⊗{\left(N_{is}\right)}^{k}\right)}^{1/j+k}\right)\\ =\frac{1}{g}\left(\overset{g}{\underset{i=1}{\sum }}{\left(\frac{2}{\left|F_{i}\right|\left(\left|F_{i}\right|+1\right)}\overset{\left|F_{i}\right|}{\underset{\lambda =1}{\sum }}\overset{\left|F_{i}\right|}{\underset{s=\lambda }{\sum }}{\left(N\right)}^{j}⊗{\left(N\right)}^{k}\right)}^{1/j+k}\right)=\frac{1}{g}\left(\overset{g}{\underset{i=1}{\sum }}{\left(\frac{2}{\left|F_{i}\right|\left(\left|F_{i}\right|+1\right)}\overset{\left|F_{i}\right|}{\underset{\lambda =1}{\sum }}\overset{\left|F_{i}\right|}{\underset{s=\lambda }{\sum }}N^{j+k}\right)}^{1/j+k}\right)\\ \frac{1}{g}\left(\overset{g}{\underset{\lambda =1}{\sum }}|N\right)=N. \end{array}, \end{array}$$

(Monotonicity) Let *M*_*λ*_=(*A*_*M*_*λ*__, *B*_*M*_*λ*__)(*λ*=1,2,…, *n*) be a set NCq-ROFNs having the same partitioned structure as *N*_*λ*_=(*A*_*N*_*λ*__, *B*_*N*_*λ*__)(*λ*=1,2,…, *n*), *A*_*M*_*λ*__ ≥ *A*_*N*_*λ*__and *B*_*M*_*λ*__ ≤ *B*_*N*_*λ*__ for all, then

(47) $$\begin{array}{c} NCq-ROFPHM^{j,k}\left(M_{1},M_{2},\ldots ,M_{\ddot{n}}\right)\geq NCq-ROFPHM^{j,k}\left(N_{1},N_{2},\ldots ,N_{\ddot{n}}\right). \end{array}$$

**Proof**

Since, *A*_*M*_*λ*__ ≥ *A*_*N*_*λ*__and *B*_*M*_*λ*__ ≤ *B*_*N*_*λ*__ for all *λ* using Definition 6, we can obtain, *M*_*λ*_ ≥ *N*_*λ*_ for all, then *A*_*M*_*iλ*__^*j*^*A*_*M*_*is*__^*k*^ ≥ *A*_*N*_*iλ*__^*j*^*A*_*is*_^*k*^ and

(48) $$\begin{array}{c} {\left(-1\right)}^{2\overset{˘}{q}+1}\left(1-{\left(1-B_{M_{i\lambda }}^{2\overset{˘}{q}}\right)}^{j}{\left(1-B_{M_{is}}^{2\overset{˘}{q}}\right)}^{k}\right)\geq {\left(-1\right)}^{2\overset{˘}{q}+1}\left(1-{\left(1-B_{N_{i\lambda }}^{2\overset{˘}{q}}\right)}^{j}{\left(1-B_{N_{is}}^{2\overset{˘}{q}}\right)}^{k}\right). \end{array}$$

Further,

(49) $$\begin{array}{c} \begin{array}{c} {℧}_{M_{i}}={\left(-1\right)}^{2\overset{˘}{q}+1}{\left(1-\Pi_{\lambda =1}^{\left|Fi\right|}\Pi_{s=\lambda }^{\left|Fi\right|}\left(1-{\left(A_{M_{i\lambda }}^{j}B_{Mi_{s}}^{k}\right)}^{2\overset{˘}{q}}\right)\right)}^{1/2q}\geq \\ {\left(-1\right)}^{2\overset{˘}{q}+1}{\left(1-\Pi_{\lambda =1}^{\left|Fi\right|}\Pi_{s=\lambda }^{\left|Fi\right|}\left(1-{\left(A_{Ni_{\lambda }}^{j}B_{N_{is}}^{k}\right)}^{2\overset{˘}{q}}\right)\right)}^{1/2q}={℧}_{N_{i}} \end{array}\text{,} \end{array}$$

and

(50) $$\begin{array}{c} \Omega_{M_{i}}={\left(-1\right)}^{2\overset{˘}{q}+1}\left(\Pi_{\lambda =1}^{\left|Fi\right|}\Pi_{s=\lambda }^{\left|Fi\right|}{\left(1-{\left(1-B_{M_{i\lambda }}^{2\overset{˘}{q}}\right)}^{j}{\left(1-B_{M_{is}}^{2\overset{˘}{q}}\right)}^{k}\right)}^{1/2q}\right)\geq \\ {\left(-1\right)}^{2\overset{˘}{q}+1}\left(\Pi_{\lambda =1}^{\left|Fi\right|}\Pi_{s=\lambda }^{\left|Fi\right|}{\left(1-{\left(1-B_{N_{i\lambda }}^{2\overset{˘}{q}}\right)}^{j}{\left(1-B_{N_{is}}^{2\overset{˘}{q}}\right)}^{k}\right)}^{1/2q}\right)=\Omega_{N_{i}}. \end{array}$$

Thus,

(51) $$\begin{array}{c} \begin{array}{c} \left(\left[\begin{array}{c} {\left(-1\right)}^{2\overset{˘}{q}+1}{\left(1-\Pi_{i=1}^{g}{\left(1-{\left(\left(1-{\left(1-{\left({℧}_{M_{i}}^{L}\right)}^{2\overset{˘}{q}}\right)}^{2/\left|F_{i}\right|\left(\left|F_{i}\right|+1\right)}\right)\right)}^{1/j+k}\right)}^{1/g}\right)}^{1/2q}\text{,}\\ {\left(-1\right)}^{2\overset{˘}{q}+1}{\left(1-\Pi_{i=1}^{g}{\left(1-{\left(\left(1-{\left(1-{\left({℧}_{M_{i}}^{U}\right)}^{2\overset{˘}{q}}\right)}^{2/\left|F_{i}\right|\left(\left|F_{i}\right|+1\right)}\right)\right)}^{1/j+k}\right)}^{1/g}\right)}^{1/2q} \end{array}\right]\right)\geq \\ \left(\left[\begin{array}{c} {\left(-1\right)}^{2\overset{˘}{q}+1}{\left(1-\Pi_{i=1}^{g}{\left(1-{\left(\left(1-{\left(1-{\left({℧}_{N_{i}}^{L}\right)}^{2\overset{˘}{q}}\right)}^{2/\left|F_{i}\right|\left(\left|F_{i}\right|+1\right)}\right)\right)}^{1/j+k}\right)}^{1/g}\right)}^{1/2q},\\ {\left(-1\right)}^{2\overset{˘}{q}+1}{\left(1-\Pi_{i=1}^{g}{\left(1-{\left(\left(1-{\left(1-{\left({℧}_{N_{i}}^{U}\right)}^{2\overset{˘}{q}}\right)}^{2/\left|F_{i}\right|\left(\left|F_{i}\right|+1\right)}\right)\right)}^{1/j+k}\right)}^{1/g}\right)}^{1/2q} \end{array}\right]\right), \end{array} \end{array}$$

and

(52) $$\begin{array}{c} \left(\left[\begin{array}{c} {\left(-1\right)}^{2\overset{˘}{q}+1}\left(\Pi_{i=1}^{g}{\left(1-{\left(1-{\left(\Omega_{M_{i}}^{L}\right)}^{4q/\left|F_{i}\right|\left(\left|F_{i}\right|+1\right)}\right)}^{1/j+k}\right)}^{1/2q*g}\right)\text{,}\\ {\left(-1\right)}^{2\overset{˘}{q}+1}\left(\Pi_{i=1}^{g}{\left(1-{\left(1-{\left(\Omega_{M_{i}}^{U}\right)}^{4q/\left|F_{i}\right|\left(\left|F_{i}\right|+1\right)}\right)}^{1/j+k}\right)}^{1/2q*g}\right) \end{array}\right]\right)\leq \\ \left(\left[\begin{array}{c} {\left(-1\right)}^{2\overset{˘}{q}+1}\left(\Pi_{i=1}^{g}{\left(1-{\left(1-{\left(\Omega_{N_{i}}^{L}\right)}^{4q/\left|F_{i}\right|\left(\left|F_{i}\right|+1\right)}\right)}^{1/j+k}\right)}^{1/2q*g}\right),\\ {\left(-1\right)}^{2\overset{˘}{q}+1}\left(\Pi_{i=1}^{g}{\left(1-{\left(1-{\left(\Omega_{N_{i}}^{U}\right)}^{4q/\left|F_{i}\right|\left(\left|F_{i}\right|+1\right)}\right)}^{1/j+k}\right)}^{1/2q*g}\right) \end{array}\right]\right). \end{array}$$

Then we use (37), we get

(53) $$\begin{array}{c} NCq-ROFPHM^{j,k}\left(M_{1},M_{2},\ldots ,M_{n}\right)\geq NCq-ROFPHM^{j,k}\left(N_{1},N_{2},\ldots ,N_{n}\right)\text{.} \end{array}$$

(Boundedness) Let *c* = 〈max_*λ*_(*A*_*N*_), min_*λ*_(*B*_*N*_)〉,*d* = 〈m*in*_*λ*_(*A*_*N*_), max_*λ*_(*B*_*N*_)〉,having a specific partition stricture *F*_*λ*_(*λ*=1,2,…, *n*). Therefore,

(54) $$\begin{array}{c} c\leq NCq-ROFPHM^{j,k}\left(N_{1},N_{2},\ldots ,N_{n}\right)\leq d. \end{array}$$

**Proof**

Since *c* = 〈max_*λ*_(*A*_*N*_), min_*λ*_(*B*_*N*_)〉,*d* = 〈min_*λ*_(*A*_*N*_), max_*λ*_(*B*_*N*_)〉,subsequently, based on the monotonicity, we have

(55) $$\begin{array}{c} NCq-ROFPHM^{j,k}\left(c,c,\ldots c\right)=c\text{,} \end{array}$$

and

(56) $$\begin{array}{c} NCq-ROFPHM^{j,k}\left(d,d,\ldots ,d\right)=d. \end{array}$$

As a result,

(57) $$\begin{array}{c} c\leq NCq-ROFPHM^{j,k}\left(N_{1},N_{2},\ldots ,N_{n}\right)\leq d\text{,} \end{array}$$

thus proved. Various particular examples of the *N*C*q* − *ROFPHM* operator can be obtained by altering the number of partitions and various values of the parameters “*j*,*k*.” The *NCq* − *ROFPHM* operator renovate into usual *NCq* − *ROFPHM* if *g*=1 as follows:

(58) $$\begin{array}{c} NCq-ROFPHM^{j,k}\left(N_{1},N_{2},\ldots ,N_{n}\right)={\left(\frac{2}{\left|F_{i}\right|\left(\left|F_{i}\right|+1\right)}\overset{\left|F_{i}\right|}{\underset{\lambda =1}{\sum }}\overset{\left|F_{i}\right|}{\underset{s=\lambda }{\sum }}N_{1\lambda }^{j}N_{1s}^{k}\right)}^{1/j+k}={\left(\frac{2}{n\left(n+1\right)}\overset{n}{\underset{\lambda =1}{\sum }}\overset{n}{\underset{s=\lambda }{\sum }}N_{\lambda }^{j}N_{s}^{k}\right)}^{1/j+k}. \end{array}$$

By giving varied values to the parameters “*j*, *k*” and *g*=1, we can clearly obtain the situations covered in equations (33)–(37).

**Definition 13 .**

Let *N*_*λ*_=(*A*_*N*_*λ*__, *B*_*N*_*λ*__)(*λ*=1,2,…, *n*) be a set of NCq-ROFNs,

*j* ≥ 0, *k* ≥ 0 and *j*+*k* ≥ 0, and *w*=(*w*_1_, *w*_2_,…, *w*_*n*_) indicate the weight vector of NCq-ROFNs *w*_*λ*_ ∈ [1,0] and ∑_*λ*=1_^*n*^*w*=1. Then NCq-ROFWPHM: [−1,0]^*n*^⟶[−1,0] such that

(59) $$\begin{array}{c} NCq-ROFWPHM_{w}^{j,k}\left(N_{1},N_{2},\ldots ,N_{n}\right)=\frac{1}{g}\left({⊕}_{i=1}^{g}{\left(\frac{2}{\left|F_{i}\right|\left(\left|F_{i}\right|+1\right)}{⊕}_{\lambda =1}^{\left|F_{i}\right|}{⊕}_{s=\lambda }^{\left|F_{i}\right|}{\left(w_{i\lambda }N_{i\lambda }\right)}^{j}⊗{\left(w_{is}N_{is}\right)}^{k}\right)}^{1/j+k}\right). \end{array}$$

**Theorem 5 .**

Let *N*_*λ*_=(*A*_*N*_*λ*__, *B*_*N*_*λ*__)(*λ*=1,2,…, *n*) be a family of NCq-ROFNs where *j* ≥ 0, *k* ≥ 0and *j*+*k* ≥ 0, and *w*=(*w*_1_, *w*_2_,…, *w*_*n*_) represents the weight vector of NCq-ROFNs, ∑_*λ*=1_^*n*^*w*=1. Then we get resultant equation by using equation (59) that is also a NCq-ROFNs given by

(60) $$\begin{array}{c} NCq-ROFWPHM_{w}^{j,k}\left(N_{1},N_{2},\ldots ,N_{n}\right)\\ \left\{\left(\begin{array}{c} \left(\begin{array}{c} \left[\begin{array}{c} {\left(-1\right)}^{2\overset{˘}{q}+1}{\left(1-\Pi_{i=1}^{g}{\left(1-{\left({\left(1-\left(1-{\left({℧}_{i}^{L}\right)}^{2\overset{˘}{q}}\right)\right)}^{2/\left|F_{i}\right|\left(\left|F_{i}\right|+1\right)}\right)}^{1/j+k}\right)}^{1/g}\right)}^{1/2q},\\ {\left(-1\right)}^{2\overset{˘}{q}+1}{\left(1-\Pi_{i=1}^{g}{\left(1-{\left({\left(1-\left(1-{\left({℧}_{i}^{U}\right)}^{2\overset{˘}{q}}\right)\right)}^{2/\left|F_{i}\right|\left(\left|F_{i}\right|+1\right)}\right)}^{1/j+k}\right)}^{1/g}\right)}^{1/2q} \end{array}\right],\\ \left[\begin{array}{c} {\left(-1\right)}^{2\overset{˘}{q}+1}\left(\Pi_{i=1}^{g}{\left(1-{\left(1-{\left(\Omega_{i}^{L}\right)}^{4q/\left|F_{i}\right|\left(\left|F_{i}\right|+1\right)}\right)}^{1/j+k}\right)}^{1/q*g}\right),\\ {\left(-1\right)}^{2\overset{˘}{q}+1}\left(\Pi_{i=1}^{g}{\left(1-{\left(1-{\left(\Omega_{i}^{L}\right)}^{4q/\left|F_{i}\right|\left(\left|F_{i}\right|+1\right)}\right)}^{1/j+k}\right)}^{1/q*g}\right) \end{array}\right] \end{array}\right),\\ \left(\begin{array}{c} {\left(-1\right)}^{2\overset{˘}{q}+1}{\left(1-\Pi_{i=1}^{g}{\left(1-{\left({\left(1-\left(1-{\left({℧}_{i}^{U}\right)}^{2\overset{˘}{q}}\right)\right)}^{2/\left|F_{i}\right|\left(\left|F_{i}\right|+1\right)}\right)}^{1/j+k}\right)}^{1/g}\right)}^{1/2q},\\ {\left(-1\right)}^{2\overset{˘}{q}+1}\left(\Pi_{i=1}^{g}{\left(1-{\left(1-{\left(\Omega_{i}^{L}\right)}^{4q/\left|F_{i}\right|\left(\left|F_{i}\right|+1\right)}\right)}^{1/j+k}\right)}^{1/q*g}\right) \end{array}\right) \end{array}\right)\right\}. \end{array}$$

where

(61) $$\begin{array}{c} {℧}_{i}^{L}={\left(-1\right)}^{2\overset{˘}{q}+1}{\left(1-\Pi_{\lambda =1}^{\left|Fi\right|}\Pi_{s=\lambda }^{\left|Fi\right|}\left(1-{\left(1-{\left(1-N_{i\lambda }^{2\overset{˘}{q}}\right)}^{w_{i\lambda }}\right)}^{j}\right)\left(1-{\left(1-{\left(1-N_{is}^{2\overset{˘}{q}}\right)}^{w_{is}}\right)}^{k}\right)\right)}^{1/2q}\text{,}\\ {℧}_{i}^{U}={\left(-1\right)}^{2\overset{˘}{q}+1}{\left(1-\Pi_{\lambda =1}^{\left|Fi\right|}\Pi_{s=\lambda }^{\left|Fi\right|}\left(1-{\left(1-{\left(1-N_{i\lambda }^{2\overset{˘}{q}}\right)}^{w_{i\lambda }}\right)}^{j}\right)\left(1-{\left(1-{\left(1-N_{is}^{2\overset{˘}{q}}\right)}^{w_{is}}\right)}^{k}\right)\right)}^{1/2q}\text{,}\\ \Omega_{i}^{L}={\left(-1\right)}^{2\overset{˘}{q}+1}\left(\Pi_{\lambda =1}^{\left|Fi\right|}\Pi_{s=\lambda }^{\left|Fi\right|}{\left(1-{\left(1-\Omega_{i\lambda }^{w_{i\lambda 2}q}\right)}^{j}{\left(1-\Omega_{is}^{w_{it2}q}\right)}^{k}\right)}^{1/2q}\right)\text{,}\\ \Omega_{i}^{U}={\left(-1\right)}^{2\overset{˘}{q}+1}\left(\Pi_{\lambda =1}^{\left|Fi\right|}\Pi_{s=\lambda }^{\left|Fi\right|}{\left(1-{\left(1-\Omega_{i\lambda }^{w_{i\lambda 2}q}\right)}^{j}{\left(1-\Omega_{is}^{w_{it2}q}\right)}^{k}\right)}^{1/2q}\right)\text{,}\\ {℧}_{i}={\left(-1\right)}^{2\overset{˘}{q}+1}{\left(1-\Pi_{\lambda =1}^{\left|Fi\right|}\Pi_{s=\lambda }^{\left|Fi\right|}\left(1-{\left(1-{\left(1-N_{i\lambda }^{2\overset{˘}{q}}\right)}^{w_{i\lambda }}\right)}^{j}\right)\left(1-{\left(1-{\left(1-N_{is}^{2\overset{˘}{q}}\right)}^{w_{is}}\right)}^{k}\right)\right)}^{1/2q}\text{,}\\ \Omega_{i}={\left(-1\right)}^{2\overset{˘}{q}+1}\left(\Pi_{\lambda =1}^{\left|Fi\right|}\Pi_{s=\lambda }^{\left|Fi\right|}{\left(1-{\left(1-\Omega_{i\lambda }^{w_{i\lambda 2}q}\right)}^{j}{\left(1-\Omega_{is}^{w_{it2}q}\right)}^{k}\right)}^{1/2q}\right)\text{.} \end{array}$$

## 4. Multi Attribute Group Decision-Making Method as an Application

In this section we will use NCq-ROFWHM and NCq-ROFWPHM operators to examine MAGDM problems, and to show their applicability with the help of NCq-ROFNs. Let $\ddot{A}=\left\{A_{1,}A_{2,}\ldots ,A_{m}\right\}$ be a set of alternatives, $C=\left\{{\overset{´}{C}}_{1,}{\overset{´}{C}}_{2,}\ldots ,{\overset{´}{C}}_{m}\right\}$ and attributes with weight vector *w* = {*w*_1,_*w*_2,_ …, *w*_*n*_}, where $w_{\tilde{ı}}\in \left[0,1\right]$ and $\sum_{\tilde{ı}=1}^{n}w_{\tilde{ı}}=1$. Let $⊼=\left\{{\overset{`}{⊼}}_{1,}{\overset{`}{⊼}}_{2,}\ldots ,{\overset{`}{⊼}}_{d}\right\}$ be a group of experts with eight vector, *ξ* = {*ξ*_1,_*ξ*_2,_ …, *ξ*_*d*_}*λ* = where *ξ*_*λ*_ ∈ [0,1] and ∑_*λ*=1_^*d*^*ξ*_*λ*_ = 1. Assume that the *λ* *th* expert provides his opinion regarding the alternatives *A*_*i*_ = {1, 2_,_ …, *m*} with regard to the qualities ${\overset{´}{C}}_{\tilde{ı}}=\left\{1,2_{,}\ldots ,m\right\}$ as a NCq-ROFNs $N_{i\tilde{ı}}^{\lambda }=\langle A_{N_{i\tilde{ı}}}^{\lambda },B_{N_{i\tilde{ı}}}^{\lambda }\rangle$.Using the expert's preference, an NCq-ROF decision matrix is created as $T_{\lambda }={\left(N_{i\tilde{ı}}^{\lambda }\right)}_{m\times n}$. Consider that there are ‘g' divisions of the set *F*_1_, *F*_2_, *F*_3_,……, *F*_*g*_ and that there is a specified connection structure between the features while keeping in mind the natural relationship structure. There is no link between qualities from different partitions and those from the same partition. The established operators are then used to address these decision-making (DM) difficulties. Algorithm steps are provided by

Step 1: To normalize the decision matrix and obtain the benefit and cost-type data. $\overset{ˇ}{T}={\overset{´}{N}}_{i\tilde{ı}}^{\lambda }={\langle A_{\overset{´}{N}i\tilde{ı}}^{\lambda },B_{{\overset{´}{N}}_{i\tilde{ı}}}^{\lambda }\rangle }_{m\times n}$ converting the value of the cost-type attributes first to the value of the benefit-type attributes, and then
  (62) $$\begin{array}{c} {\overset{´}{N}}_{i\tilde{ı}}^{\lambda }=\left(\begin{array}{c} N_{i\tilde{ı}}^{\lambda }\text{ for benefit}-\text{type attribute of}{\;}_{\tilde{ı}}^{C}\;\\ {\left(N_{i\tilde{ı}}^{\lambda }\right)}^{c}\text{for cost}-\text{type attribute of}{\;}_{\tilde{ı}}^{C} \end{array}\right). \end{array}$$
where ${\left(N_{i\tilde{ı}}^{\lambda }\right)}^{c}=\langle B_{N_{i\tilde{ı}}}^{\lambda },A_{N_{i\tilde{ı}}}^{\lambda }\rangle$.
Step 2: To aggregate all the normalized data. ${\overset{ˇ}{T}}_{\lambda }$= (*λ* = 1,2,3,…, *d*) into a collective DM $M={\left[V_{i\tilde{ı}}\right]}_{m\times n}={\langle A_{{\overset{´}{N}}_{i\tilde{ı}}}^{\lambda },B_{{\overset{´}{N}}_{i\tilde{ı}}}^{\lambda }\rangle }_{m\times n}$.
  (63) $$\begin{array}{c} V_{ij}=NCq-ROFWHM_{\xi }^{j,k}\left({\overset{´}{N}}_{i\tilde{ı}}^{1},{\overset{´}{N}}_{i\tilde{ı}}^{2},{\overset{´}{N}}_{i\tilde{ı}}^{3},\ldots ,{\overset{´}{N}}_{i\tilde{ı}}^{d}\right)\\ \left\{\begin{array}{c} \left(\begin{array}{c} \left[\begin{array}{c} {\left(-1\right)}^{2\overset{˘}{q}+1}{\left(1-\Pi_{\lambda =1}^{n}\Pi_{s=\lambda }^{n}{\left(1-{\left({℧}_{N_{\lambda }}^{L}\right)}^{2\overset{˘}{q}}\right)}^{2/n\left(n+1\right)}\right)}^{1/2\overset{˘}{q}\left(j+k\right)},\\ {\left(-1\right)}^{2\overset{˘}{q}+1}{\left(1-\Pi_{\lambda =1}^{n}\Pi_{s=\lambda }^{n}{\left(1-{\left({℧}_{N_{\lambda }}^{U}\right)}^{2\overset{˘}{q}}\right)}^{2/n\left(n+1\right)}\right)}^{1/2\overset{˘}{q}\left(j+k\right)} \end{array}\right],\\ \left[\begin{array}{c} {\left(-1\right)}^{2\overset{˘}{q}+1}{\left(1-{\left(1-\Pi_{\lambda =1}^{n}\Pi_{s=\lambda }^{n}{\left(\Omega_{N_{\lambda }}^{L}\right)}^{2\overset{˘}{q}/n\left(n+1\right)}\right)}^{1/j+k}\right)}^{1/2q}\\ {\left(-1\right)}^{2\overset{˘}{q}+1}{\left(1-{\left(1-\Pi_{\lambda =1}^{n}\Pi_{s=\lambda }^{n}{\left(\Omega_{N_{\lambda }}^{U}\right)}^{2\overset{˘}{q}/n\left(n+1\right)}\right)}^{1/j+k}\right)}^{1/2q} \end{array}\right] \end{array}\right),\\ \left(\begin{array}{c} {\left(-1\right)}^{2\overset{˘}{q}+1}{\left(1-\Pi_{\lambda =1}^{n}\Pi_{s=\lambda }^{n}{\left(1-{\left({℧}_{N_{\lambda }}\right)}^{2\overset{˘}{q}}\right)}^{2/n\left(n+1\right)}\right)}^{1/2\overset{˘}{q}\left(j+k\right)},\\ {\left(-1\right)}^{2\overset{˘}{q}+1}{\left(1-{\left(1-\Pi_{\lambda =1}^{n}\Pi_{s=\lambda }^{n}{\left(\Omega_{N_{\lambda }}\right)}^{2\overset{˘}{q}/n\left(n+1\right)}\right)}^{1/2\left(j+k\right)}\right)}^{1/2q} \end{array}\right), \end{array}\right\}, \end{array}$$
where
  (64) $$\begin{array}{c} \left[{℧}_{\lambda }^{L},\left({℧}_{\lambda }^{U}\right)\right]=\left[\begin{array}{c} {\left(-1\right)}^{2\overset{˘}{q}+1}\left({\left(1-{\left(1-{\left({℧}_{\lambda }^{L}\right)}^{2\overset{˘}{q}}\right)}^{B_{\lambda }}\right)}^{j/2\overset{˘}{q}}{\left(1-{\left(1-{\left({℧}_{s}^{L}\right)}^{2\overset{˘}{q}}\right)}^{B_{s}}\right)}^{k/2\overset{˘}{q}}\right)\text{,}\\ {\left(-1\right)}^{2\overset{˘}{q}+1}\left({\left(1-{\left(1-{\left({℧}_{\lambda }^{U}\right)}^{2\overset{˘}{q}}\right)}^{B_{\lambda }}\right)}^{j/2\overset{˘}{q}}{\left(1-{\left(1-{\left({℧}_{s}^{U}\right)}^{2\overset{˘}{q}}\right)}^{B_{s}}\right)}^{k/2\overset{˘}{q}}\right)\text{,} \end{array}\right],\\ \left[\Omega_{\lambda }^{L},\Omega_{\lambda }^{U}\right]=\left[\begin{array}{c} {\left(-1\right)}^{2\overset{˘}{q}+1}\left({\left(1-{\left(1-{\left(\Omega_{\lambda }^{L}\right)}^{2\overset{˘}{q}B_{\lambda }}\right)}^{j}{\left(1-{\left(\Omega_{s}^{L}\right)}^{2\overset{˘}{q}B_{t}}\right)}^{k}\right)}^{j/2\overset{˘}{q}}\right)\text{,}\\ {\left(-1\right)}^{2\overset{˘}{q}+1}\left({\left(1-{\left(1-{\left(\Omega_{\lambda }^{U}\right)}^{2\overset{˘}{q}B_{\lambda }}\right)}^{j}{\left(1-{\left(\Omega_{s}^{U}\right)}^{2\overset{˘}{q}B_{t}}\right)}^{k}\right)}^{j/2\overset{˘}{q}}\right) \end{array}\right],\\ {℧}_{\lambda }^{L}={\left(-1\right)}^{2\overset{˘}{q}+1}\left({\left(1-{\left(1-{\left({℧}_{\lambda }\right)}^{2\overset{˘}{q}}\right)}^{B_{\lambda }}\right)}^{j/2\overset{˘}{q}}{\left(1-{\left(1-{\left({℧}_{s}\right)}^{2\overset{˘}{q}}\right)}^{B_{s}}\right)}^{k/2\overset{˘}{q}}\right),\\ \Omega_{\lambda }^{L}={\left(-1\right)}^{2\overset{˘}{q}+1}\left({\left(1-{\left(1-{\left(\Omega_{\lambda }\right)}^{2\overset{˘}{q}B_{\lambda }}\right)}^{j}{\left(1-{\left(\Omega_{s}\right)}^{2\overset{˘}{q}B_{t}}\right)}^{k}\right)}^{j/2\overset{˘}{q}}\right). \end{array}$$
Step 3: Assume a division form among the attributes to arrive at the collective assessment values. $V_{i}=\left(\langle A_{\overset{´}{N}i\tilde{ı}}^{\lambda },B_{{\overset{´}{N}}_{i\tilde{ı}}}^{\lambda }\rangle \right)\left(i=1,2,3,\ldots m\right);\left(\tilde{ı}=1,2,3,\ldots n\right)$ of alternatives *A*_*i*_.
  (65) $$\begin{array}{c} V_{i}=NCQ-ROFWHP_{w}^{j,k}\left(V_{i1}V_{i2},\ldots ,V_{in}\right). \end{array}$$
Step 4: To find score values $\hat{S}\left(V_{i}\right)$ of each alternative *A*(*i* = 1,2,3,…, *m*).

**Example 2 .**

In this section we provide a brief overview of the outcomes of a brand-new technique and show its efficacy. Utilizing the full potential of mobile apps for online education, business administrators can check the effectiveness of these programs. Four possibilities have been suggested as possible options in the beginning stages. Moodle A_1_, LMS A_2_, Zoom A_3_, and NoonA_4_ are the four applications. There are four experts on the judgment board, [E1, E2, E3, E4] each with a different area of competence. Take into account that *λ* represents the different expert weights, or *λ*=(0.03,0.1,0.27,0.6). The five interconnected characteristics listed by the assessment committee are as follows: the app's download, data storage speeds, data loading speed in and battery use (C1an dC 2, C3 and C4, respectively). Assume represents different attribute weights, for example, w=(0.17,0.2,0.23,0.4). The two subsets of the five qualities are separated based on how they relate to one another fundamentally. F_1_={C_1_, C_3_, C_5_}, F_1_={C_2_, C_4_}. Data in the form of NCq-ROFNs must be submitted by experts for examination. The expert assessment statistics are displayed in Tables 1–4, and E_i_=(i=1,2,3,4).

  Step 1: Given that *C*_3_ is a cost-type attribute, we can normalize the decision-making data using equation (62). The normalized data is displayed in Tables 5–8.
  Step 2: To obtain the entire decision matrix, use equation (63). $M={\left\{{\tilde{U}}_{i\tilde{ı}}\right\}}_{4\times 5}={\left\{\langle A_{{\tilde{U}}_{i\tilde{ı}}},B_{{\tilde{U}}_{i\tilde{ı}}}\rangle \right\}}_{4\times 5}$. Additionally, we set the parameters *j* = 1, *k* = 1, and *q* = 3 to be true. This MAGDM seeks to identify the best choice. The complete NCq-ROF decision matrix *M* is shown in Table 9.
  STEP 3: Use (23) to calculate all of the evaluation values for each option, then use *A*_*i*_ and ${\tilde{U}}_{i}$ to obtain the values for each alternative's *A*_*i*_(*i*=1,2,3,4) collective evaluation.
 
${\tilde{U}}_{1}=\left(\left[-.0000754307,-.0039453\right],\left[-.836279,-.827616\right],\left(-.00345878,-.865973\right)\right)$, ${\tilde{U}}_{2}=\left(\left[-.0000856423,-.0054665\right],\left[-.839751,-.829231\right],\left(-.00265612,-.860356\right)\right)$, ${\tilde{U}}_{3}=\left(\left[-.0000346567,-.0039675\right],\left[-.836134,-.826964\right],\left(-.00467348,-.863867\right)\right)$, ${\tilde{U}}_{4}=\left(\left[-.0000126569,-.0067831\right],\left[-.830651,-.825320\right],\left(-.00679601,-.865328\right)\right)$.
  STEP 4: We compute score values $S\left({\tilde{U}}_{i}\right)$of ${\tilde{U}}_{i}$ as follows: $S\left({\tilde{U}}_{1}\right)=-.57679527,S\left({\tilde{U}}_{2}\right)=-.5976312,S\left({\tilde{U}}_{3}\right)=-.56140327,S\left({\tilde{U}}_{4}\right)=0.5787565$ as $S\left({\tilde{U}}_{3}\right)>S\left({\tilde{U}}_{1}\right)>S\left({\tilde{U}}_{4}\right)>S\left({\tilde{U}}_{2}\right)$.

Hence *A*_3_ > *A*_1_ > *A*_4_ > *A*_2_ and *A*_3_ is best alternative.The Influence of the parameter Values on the Ranking Results. In the following section, we will investigate how the parameters *q*, *j*, and *k* impact the findings of the alternatives. Put *j*=1, *k*=1 and *q*=3 in the previous computing technique for our convenience and without losing generality. From Table 10, it is clear that the ranking outcomes for the scenarios *q*=4,5,7,8 and *A*_3_ > *A*_1_ > *A*_4_ > *A*_2_ are identical. Thus the ranking outcomes are shown as in Figure 1, and finally, we can say that the other top options remain the same when the parameter's value changes.

These are different from the results obtained for j=0 and k=1 having ranking results A_4_ > A_1_ > A_2_ > A_3_. As a result, it is possible to obtain varied ranking results by varying the values of the parameters *j* and *k*. If one parameter is fixed and the other is changed, the score and ranking results may change, as shown in Table 11. We can observe that the values of the parameters *j* and *k* affect the ranking outcomes, as shown in Figure 2.

## 5. Conclusion

In this study, we focus on the structure of N-cubic q-rung orthopair fuzzy sets. The score function under R-order and the comparison rule for two N-cubic q-rung orthopair fuzzy sets also define some aggregation operators, i.e., N-cubic q-rung orthopair fuzzy Hamy mean operator, N-cubic q-rung orthopair fuzzy weighted Hamy mean operator, N-cubic q-rung orthopair fuzzy power Hamy mean operator, and N-cubic q-rung orthopair fuzzy power weighted Hamy mean operator. N-structure can enhance decision-making performance. The recently discovered N-cubic q-ROFSs, which combine NQ-ROFSs and NIVqRFSs into a single structure, allow decision-makers greater space to work on multi-attribute group decision-making problems. As a result of the debate, we have discussed specific instances of the operators and created a method for solving MAGDM problems using NCq-ROFNs. In this study we analyze the use of mobile app in the education sector. Further research, problem-solving, and decision-making are possible to solve, and other operators may be able to be created through this method. In future someone can apply the N-cubic q-rung orthopair fuzzy sets in different decision-making technique.

## Figures and Tables

**Figure 1:** Ranking result for *q* = 4,5,7,8.

**Figure 2:** Ranking result for various values of parameters j and k.

**Table 1:** For NCq-ROFDM of Q_1_.

	*C*_1_	*C*_2_	*C*_3_	*C*_4_	*C*_5_
*A*_1_	$\left(\left(\begin{array}{c} \left[\begin{array}{cc} -6 & -3 \end{array}\right]\\ \left[\begin{array}{cc} -5 & -4 \end{array}\right]\\ \left[\begin{array}{cc} -6 & -1 \end{array}\right] \end{array}\right)\right)$	$\left(\left(\begin{array}{c} \left[\begin{array}{cc} -7 & -3 \end{array}\right]\\ \left[\begin{array}{cc} -5 & -4 \end{array}\right]\\ \left[\begin{array}{cc} -9 & -4 \end{array}\right] \end{array}\right)\right)$	$\left(\left(\begin{array}{c} \left[\begin{array}{cc} -7 & -3 \end{array}\right]\\ \left[\begin{array}{cc} -5 & -4 \end{array}\right]\\ \left[\begin{array}{cc} -9 & -4 \end{array}\right] \end{array}\right)\right)$	$\left(\left(\begin{array}{c} \left[\begin{array}{cc} -9 & -6 \end{array}\right]\\ \left[\begin{array}{cc} -5 & -5 \end{array}\right]\\ \left[\begin{array}{cc} -4 & -1 \end{array}\right] \end{array}\right)\right)$	$\left(\left(\begin{array}{c} \left[\begin{array}{cc} -2 & -2 \end{array}\right]\\ \left[\begin{array}{cc} -9 & -5 \end{array}\right]\\ \left[\begin{array}{cc} -9 & -7 \end{array}\right] \end{array}\right)\right)$
*A*_2_	$\left(\left(\begin{array}{c} \left[\begin{array}{cc} -8 & -5 \end{array}\right]\\ \left[\begin{array}{cc} -7 & -6 \end{array}\right]\\ \left[\begin{array}{cc} -4 & -3 \end{array}\right] \end{array}\right)\right)$	$\left(\left(\begin{array}{c} \left[\begin{array}{cc} -6 & -2 \end{array}\right]\\ \left[\begin{array}{cc} -6 & -5 \end{array}\right]\\ \left[\begin{array}{cc} -6 & -1 \end{array}\right] \end{array}\right)\right)$	$\left(\left(\begin{array}{c} \left[\begin{array}{cc} -8 & -5 \end{array}\right]\\ \left[\begin{array}{cc} -6 & -3 \end{array}\right]\\ \left[\begin{array}{cc} -6 & -3 \end{array}\right] \end{array}\right)\right)$	$\left(\left(\begin{array}{c} \left[\begin{array}{cc} -6 & -2 \end{array}\right]\\ \left[\begin{array}{cc} -8 & -6 \end{array}\right]\\ \left[\begin{array}{cc} -6 & -3 \end{array}\right] \end{array}\right)\right)$	$\left(\left(\begin{array}{c} \left[\begin{array}{cc} -7 & -2 \end{array}\right]\\ \left[\begin{array}{cc} -4 & -5 \end{array}\right]\\ \left[\begin{array}{cc} -7 & -1 \end{array}\right] \end{array}\right)\right)$
*A*_3_	$\left(\left(\begin{array}{c} \left[\begin{array}{cc} -3 & -2 \end{array}\right]\\ \left[\begin{array}{cc} -5 & -5 \end{array}\right]\\ \left[\begin{array}{cc} -9 & -6 \end{array}\right] \end{array}\right)\right)$	$\left(\left(\begin{array}{c} \left[\begin{array}{cc} -6 & -5 \end{array}\right]\\ \left[\begin{array}{cc} -7 & -4 \end{array}\right]\\ \left[\begin{array}{cc} -6 & -1 \end{array}\right] \end{array}\right)\right)$	$\left(\left(\begin{array}{c} \left[\begin{array}{cc} -7 & -6 \end{array}\right]\\ \left[\begin{array}{cc} -7 & -4 \end{array}\right]\\ \left[\begin{array}{cc} -9 & -8 \end{array}\right] \end{array}\right)\right)$	$\left(\left(\begin{array}{c} \left[\begin{array}{cc} -8 & -6 \end{array}\right]\\ \left[\begin{array}{cc} -5 & -5 \end{array}\right]\\ \left[\begin{array}{cc} -6 & -4 \end{array}\right] \end{array}\right)\right)$	$\left(\left(\begin{array}{c} \left[\begin{array}{cc} -9 & -8 \end{array}\right]\\ \left[\begin{array}{cc} -6 & -5 \end{array}\right]\\ \left[\begin{array}{cc} -7 & -1 \end{array}\right] \end{array}\right)\right)$
*A*_4_	$\left(\left(\begin{array}{c} \left[\begin{array}{cc} -4 & -2 \end{array}\right]\\ \left[\begin{array}{cc} -8 & -5 \end{array}\right]\\ \left[\begin{array}{cc} -8 & -7 \end{array}\right] \end{array}\right)\right)$	$\left(\left(\begin{array}{c} \left[\begin{array}{cc} -9 & -4 \end{array}\right]\\ \left[\begin{array}{cc} -7 & -5 \end{array}\right]\\ \left[\begin{array}{cc} -6 & -6 \end{array}\right] \end{array}\right)\right)$	$\left(\left(\begin{array}{c} \left[\begin{array}{cc} -8 & -7 \end{array}\right]\\ \left[\begin{array}{cc} -6 & -5 \end{array}\right]\\ \left[\begin{array}{cc} -7 & -4 \end{array}\right] \end{array}\right)\right)$	$\left(\left(\begin{array}{c} \left[\begin{array}{cc} -6 & -2 \end{array}\right]\\ \left[\begin{array}{cc} -9 & -5 \end{array}\right]\\ \left[\begin{array}{cc} -5 & -4 \end{array}\right] \end{array}\right)\right)$	$\left(\left(\begin{array}{c} \left[\begin{array}{cc} -7 & -5 \end{array}\right]\\ \left[\begin{array}{cc} -6 & -4 \end{array}\right]\\ \left[\begin{array}{cc} -9 & -3 \end{array}\right] \end{array}\right)\right)$

**Table 2:** For NCq-ROFDM of Q_2_.

	*C*_1_	*C*_2_	*C*_3_	*C*_4_	*C*_5_
*A*_1_	$\left(\left(\begin{array}{c} \left[\begin{array}{cc} -5 & -4 \end{array}\right]\\ \left[\begin{array}{cc} -7 & -5 \end{array}\right]\\ \left[\begin{array}{cc} -7 & -2 \end{array}\right] \end{array}\right)\right)$	$\left(\left(\begin{array}{c} \left[\begin{array}{cc} -7 & -6 \end{array}\right]\\ \left[\begin{array}{cc} -3 & -2 \end{array}\right]\\ \left[\begin{array}{cc} -3 & -8 \end{array}\right] \end{array}\right)\right)$	$\left(\left(\begin{array}{c} \left[\begin{array}{cc} -5 & -3 \end{array}\right]\\ \left[\begin{array}{cc} -6 & -4 \end{array}\right]\\ \left[\begin{array}{cc} -6 & -8 \end{array}\right] \end{array}\right)\right)$	$\left(\left(\begin{array}{c} \left[\begin{array}{cc} -4 & -3 \end{array}\right]\\ \left[\begin{array}{cc} -3 & -2 \end{array}\right]\\ \left[\begin{array}{cc} -1 & -4 \end{array}\right] \end{array}\right)\right)$	$\left(\left(\begin{array}{c} \left[\begin{array}{cc} -6 & -3 \end{array}\right]\\ \left[\begin{array}{cc} -4 & -2 \end{array}\right]\\ \left[\begin{array}{cc} -8 & -1 \end{array}\right] \end{array}\right)\right)$
*A*_2_	$\left(\left(\begin{array}{c} \left[\begin{array}{cc} -3 & -2 \end{array}\right]\\ \left[\begin{array}{cc} -5 & -4 \end{array}\right]\\ \left[\begin{array}{cc} -8 & -2 \end{array}\right] \end{array}\right)\right)$	$\left(\left(\begin{array}{c} \left[\begin{array}{cc} -2 & -1 \end{array}\right]\\ \left[\begin{array}{cc} -7 & -6 \end{array}\right]\\ \left[\begin{array}{cc} -9 & -4 \end{array}\right] \end{array}\right)\right)$	$\left(\left(\begin{array}{c} \left[\begin{array}{cc} -7 & -5 \end{array}\right]\\ \left[\begin{array}{cc} -4 & -3 \end{array}\right]\\ \left[\begin{array}{cc} -5 & -8 \end{array}\right] \end{array}\right)\right)$	$\left(\left(\begin{array}{c} \left[\begin{array}{cc} -7 & -6 \end{array}\right]\\ \left[\begin{array}{cc} -2 & -1 \end{array}\right]\\ \left[\begin{array}{cc} -6 & -3 \end{array}\right] \end{array}\right)\right)$	$\left(\left(\begin{array}{c} \left[\begin{array}{cc} -2 & -1 \end{array}\right]\\ \left[\begin{array}{cc} -5 & -4 \end{array}\right]\\ \left[\begin{array}{cc} -7 & -4 \end{array}\right] \end{array}\right)\right)$
*A*_3_	$\left(\left(\begin{array}{c} \left[\begin{array}{cc} -9 & -7 \end{array}\right]\\ \left[\begin{array}{cc} -2 & -1 \end{array}\right]\\ \left[\begin{array}{cc} -6 & -1 \end{array}\right] \end{array}\right)\right)$	$\left(\left(\begin{array}{c} \left[\begin{array}{cc} -9 & -7 \end{array}\right]\\ \left[\begin{array}{cc} -2 & -1 \end{array}\right]\\ \left[\begin{array}{cc} -6 & -2 \end{array}\right] \end{array}\right)\right)$	$\left(\left(\begin{array}{c} \left[\begin{array}{cc} -8 & -6 \end{array}\right]\\ \left[\begin{array}{cc} -7 & -3 \end{array}\right]\\ \left[\begin{array}{cc} -8 & -5 \end{array}\right] \end{array}\right)\right)$	$\left(\left(\begin{array}{c} \left[\begin{array}{cc} -6 & -5 \end{array}\right]\\ \left[\begin{array}{cc} -7 & -5 \end{array}\right]\\ \left[\begin{array}{cc} -9 & -2 \end{array}\right] \end{array}\right)\right)$	$\left(\left(\begin{array}{c} \left[\begin{array}{cc} -6 & -4 \end{array}\right]\\ \left[\begin{array}{cc} -3 & -2 \end{array}\right]\\ \left[\begin{array}{cc} -6 & -5 \end{array}\right] \end{array}\right)\right)$
*A*_4_	$\left(\left(\begin{array}{c} \left[\begin{array}{cc} -5 & -3 \end{array}\right]\\ \left[\begin{array}{cc} -6 & -4 \end{array}\right]\\ \left[\begin{array}{cc} -7 & -4 \end{array}\right] \end{array}\right)\right)$	$\left(\left(\begin{array}{c} \left[\begin{array}{cc} -3 & -2 \end{array}\right]\\ \left[\begin{array}{cc} -8 & -5 \end{array}\right]\\ \left[\begin{array}{cc} -6 & -4 \end{array}\right] \end{array}\right)\right)$	$\left(\left(\begin{array}{c} \left[\begin{array}{cc} -6 & -5 \end{array}\right]\\ \left[\begin{array}{cc} -5 & -5 \end{array}\right]\\ \left[\begin{array}{cc} -5 & -3 \end{array}\right] \end{array}\right)\right)$	$\left(\left(\begin{array}{c} \left[\begin{array}{cc} -8 & -7 \end{array}\right]\\ \left[\begin{array}{cc} -9 & -5 \end{array}\right]\\ \left[\begin{array}{cc} -5 & -4 \end{array}\right] \end{array}\right)\right)$	$\left(\left(\begin{array}{c} \left[\begin{array}{cc} -4 & -2 \end{array}\right]\\ \left[\begin{array}{cc} -3 & -2 \end{array}\right]\\ \left[\begin{array}{cc} -5 & -4 \end{array}\right] \end{array}\right)\right)$

**Table 3:** For NCq-ROFDM of *Q*_3_.

	*C*_1_	*C*_2_	*C*_3_	*C*_4_	*C*_5_
*A*_1_	$\left(\left(\begin{array}{c} \left[\begin{array}{cc} -5 & -4 \end{array}\right]\\ \left[\begin{array}{cc} -7 & -5 \end{array}\right]\\ \left[\begin{array}{cc} -7 & -2 \end{array}\right] \end{array}\right)\right)$	$\left(\left(\begin{array}{c} \left[\begin{array}{cc} -7 & -6 \end{array}\right]\\ \left[\begin{array}{cc} -3 & -2 \end{array}\right]\\ \left[\begin{array}{cc} -3 & -8 \end{array}\right] \end{array}\right)\right)$	$\left(\left(\begin{array}{c} \left[\begin{array}{cc} -5 & -3 \end{array}\right]\\ \left[\begin{array}{cc} -6 & -4 \end{array}\right]\\ \left[\begin{array}{cc} -6 & -8 \end{array}\right] \end{array}\right)\right)$	$\left(\left(\begin{array}{c} \left[\begin{array}{cc} -4 & -3 \end{array}\right]\\ \left[\begin{array}{cc} -3 & -2 \end{array}\right]\\ \left[\begin{array}{cc} -1 & -4 \end{array}\right] \end{array}\right)\right)$	$\left(\left(\begin{array}{c} \left[\begin{array}{cc} -6 & -3 \end{array}\right]\\ \left[\begin{array}{cc} -4 & -2 \end{array}\right]\\ \left[\begin{array}{cc} -8 & -1 \end{array}\right] \end{array}\right)\right)$
*A*_2_	$\left(\left(\begin{array}{c} \left[\begin{array}{cc} -3 & -2 \end{array}\right]\\ \left[\begin{array}{cc} -5 & -4 \end{array}\right]\\ \left[\begin{array}{cc} -8 & -2 \end{array}\right] \end{array}\right)\right)$	$\left(\left(\begin{array}{c} \left[\begin{array}{cc} -2 & -1 \end{array}\right]\\ \left[\begin{array}{cc} -7 & -6 \end{array}\right]\\ \left[\begin{array}{cc} -9 & -4 \end{array}\right] \end{array}\right)\right)$	$\left(\left(\begin{array}{c} \left[\begin{array}{cc} -7 & -5 \end{array}\right]\\ \left[\begin{array}{cc} -4 & -3 \end{array}\right]\\ \left[\begin{array}{cc} -5 & -8 \end{array}\right] \end{array}\right)\right)$	$\left(\left(\begin{array}{c} \left[\begin{array}{cc} -7 & -6 \end{array}\right]\\ \left[\begin{array}{cc} -2 & -1 \end{array}\right]\\ \left[\begin{array}{cc} -6 & -3 \end{array}\right] \end{array}\right)\right)$	$\left(\left(\begin{array}{c} \left[\begin{array}{cc} -2 & -1 \end{array}\right]\\ \left[\begin{array}{cc} -5 & -4 \end{array}\right]\\ \left[\begin{array}{cc} -7 & -4 \end{array}\right] \end{array}\right)\right)$
*A*_3_	$\left(\left(\begin{array}{c} \left[\begin{array}{cc} -9 & -7 \end{array}\right]\\ \left[\begin{array}{cc} -2 & -1 \end{array}\right]\\ \left[\begin{array}{cc} -6 & -1 \end{array}\right] \end{array}\right)\right)$	$\left(\left(\begin{array}{c} \left[\begin{array}{cc} -9 & -7 \end{array}\right]\\ \left[\begin{array}{cc} -2 & -1 \end{array}\right]\\ \left[\begin{array}{cc} -6 & -2 \end{array}\right] \end{array}\right)\right)$	$\left(\left(\begin{array}{c} \left[\begin{array}{cc} -8 & -6 \end{array}\right]\\ \left[\begin{array}{cc} -7 & -3 \end{array}\right]\\ \left[\begin{array}{cc} -8 & -5 \end{array}\right] \end{array}\right)\right)$	$\left(\left(\begin{array}{c} \left[\begin{array}{cc} -6 & -5 \end{array}\right]\\ \left[\begin{array}{cc} -7 & -5 \end{array}\right]\\ \left[\begin{array}{cc} -9 & -2 \end{array}\right] \end{array}\right)\right)$	$\left(\left(\begin{array}{c} \left[\begin{array}{cc} -6 & -4 \end{array}\right]\\ \left[\begin{array}{cc} -3 & -2 \end{array}\right]\\ \left[\begin{array}{cc} -6 & -5 \end{array}\right] \end{array}\right)\right)$
*A*_4_	$\left(\left(\begin{array}{c} \left[\begin{array}{cc} -5 & -3 \end{array}\right]\\ \left[\begin{array}{cc} -6 & -4 \end{array}\right]\\ \left[\begin{array}{cc} -7 & -4 \end{array}\right] \end{array}\right)\right)$	$\left(\left(\begin{array}{c} \left[\begin{array}{cc} -3 & -2 \end{array}\right]\\ \left[\begin{array}{cc} -8 & -5 \end{array}\right]\\ \left[\begin{array}{cc} -6 & -4 \end{array}\right] \end{array}\right)\right)$	$\left(\left(\begin{array}{c} \left[\begin{array}{cc} -6 & -5 \end{array}\right]\\ \left[\begin{array}{cc} -5 & -5 \end{array}\right]\\ \left[\begin{array}{cc} -5 & -3 \end{array}\right] \end{array}\right)\right)$	$\left(\left(\begin{array}{c} \left[\begin{array}{cc} -8 & -7 \end{array}\right]\\ \left[\begin{array}{cc} -9 & -5 \end{array}\right]\\ \left[\begin{array}{cc} -5 & -4 \end{array}\right] \end{array}\right)\right)$	$\left(\left(\begin{array}{c} \left[\begin{array}{cc} -4 & -2 \end{array}\right]\\ \left[\begin{array}{cc} -3 & -2 \end{array}\right]\\ \left[\begin{array}{cc} -5 & -4 \end{array}\right] \end{array}\right)\right)$

**Table 4:** For NCq-ROFDM of *Q*_4_.

	*C*_1_	*C*_2_	*C*_3_	*C*_4_	*C*_5_
*A*_1_	$\left(\left(\begin{array}{c} \left[\begin{array}{cc} -6 & -3 \end{array}\right]\\ \left[\begin{array}{cc} -5 & -4 \end{array}\right]\\ \left[\begin{array}{cc} -6 & -1 \end{array}\right] \end{array}\right)\right)$	$\left(\left(\begin{array}{c} \left[\begin{array}{cc} -7 & -3 \end{array}\right]\\ \left[\begin{array}{cc} -5 & -4 \end{array}\right]\\ \left[\begin{array}{cc} -9 & -4 \end{array}\right] \end{array}\right)\right)$	$\left(\left(\begin{array}{c} \left[\begin{array}{cc} -7 & -3 \end{array}\right]\\ \left[\begin{array}{cc} -5 & -4 \end{array}\right]\\ \left[\begin{array}{cc} -9 & -4 \end{array}\right] \end{array}\right)\right)$	$\left(\left(\begin{array}{c} \left[\begin{array}{cc} -9 & -6 \end{array}\right]\\ \left[\begin{array}{cc} -5 & -5 \end{array}\right]\\ \left[\begin{array}{cc} -4 & -1 \end{array}\right] \end{array}\right)\right)$	$\left(\left(\begin{array}{c} \left[\begin{array}{cc} -2 & -2 \end{array}\right]\\ \left[\begin{array}{cc} -9 & -5 \end{array}\right]\\ \left[\begin{array}{cc} -9 & -7 \end{array}\right] \end{array}\right)\right)$
*A*_2_	$\left(\left(\begin{array}{c} \left[\begin{array}{cc} -8 & -5 \end{array}\right]\\ \left[\begin{array}{cc} -7 & -6 \end{array}\right]\\ \left[\begin{array}{cc} -4 & -3 \end{array}\right] \end{array}\right)\right)$	$\left(\left(\begin{array}{c} \left[\begin{array}{cc} -6 & -2 \end{array}\right]\\ \left[\begin{array}{cc} -6 & -5 \end{array}\right]\\ \left[\begin{array}{cc} -6 & -1 \end{array}\right] \end{array}\right)\right)$	$\left(\left(\begin{array}{c} \left[\begin{array}{cc} -8 & -5 \end{array}\right]\\ \left[\begin{array}{cc} -6 & -3 \end{array}\right]\\ \left[\begin{array}{cc} -6 & -3 \end{array}\right] \end{array}\right)\right)$	$\left(\left(\begin{array}{c} \left[\begin{array}{cc} -6 & -2 \end{array}\right]\\ \left[\begin{array}{cc} -8 & -6 \end{array}\right]\\ \left[\begin{array}{cc} -6 & -3 \end{array}\right] \end{array}\right)\right)$	$\left(\left(\begin{array}{c} \left[\begin{array}{cc} -7 & -2 \end{array}\right]\\ \left[\begin{array}{cc} -4 & -5 \end{array}\right]\\ \left[\begin{array}{cc} -7 & -1 \end{array}\right] \end{array}\right)\right)$
*A*_3_	$\left(\left(\begin{array}{c} \left[\begin{array}{cc} -3 & -2 \end{array}\right]\\ \left[\begin{array}{cc} -5 & -5 \end{array}\right]\\ \left[\begin{array}{cc} -9 & -6 \end{array}\right] \end{array}\right)\right)$	$\left(\left(\begin{array}{c} \left[\begin{array}{cc} -6 & -5 \end{array}\right]\\ \left[\begin{array}{cc} -7 & -4 \end{array}\right]\\ \left[\begin{array}{cc} -6 & -1 \end{array}\right] \end{array}\right)\right)$	$\left(\left(\begin{array}{c} \left[\begin{array}{cc} -7 & -6 \end{array}\right]\\ \left[\begin{array}{cc} -7 & -4 \end{array}\right]\\ \left[\begin{array}{cc} -9 & -8 \end{array}\right] \end{array}\right)\right)$	$\left(\left(\begin{array}{c} \left[\begin{array}{cc} -8 & -6 \end{array}\right]\\ \left[\begin{array}{cc} -5 & -5 \end{array}\right]\\ \left[\begin{array}{cc} -6 & -4 \end{array}\right] \end{array}\right)\right)$	$\left(\left(\begin{array}{c} \left[\begin{array}{cc} -9 & -8 \end{array}\right]\\ \left[\begin{array}{cc} -6 & -5 \end{array}\right]\\ \left[\begin{array}{cc} -7 & -1 \end{array}\right] \end{array}\right)\right)$
*A*_4_	$\left(\left(\begin{array}{c} \left[\begin{array}{cc} -4 & -2 \end{array}\right]\\ \left[\begin{array}{cc} -8 & -5 \end{array}\right]\\ \left[\begin{array}{cc} -8 & -7 \end{array}\right] \end{array}\right)\right)$	$\left(\left(\begin{array}{c} \left[\begin{array}{cc} -9 & -4 \end{array}\right]\\ \left[\begin{array}{cc} -7 & -5 \end{array}\right]\\ \left[\begin{array}{cc} -6 & -6 \end{array}\right] \end{array}\right)\right)$	$\left(\left(\begin{array}{c} \left[\begin{array}{cc} -8 & -7 \end{array}\right]\\ \left[\begin{array}{cc} -6 & -5 \end{array}\right]\\ \left[\begin{array}{cc} -7 & -4 \end{array}\right] \end{array}\right)\right)$	$\left(\left(\begin{array}{c} \left[\begin{array}{cc} -6 & -2 \end{array}\right]\\ \left[\begin{array}{cc} -9 & -5 \end{array}\right]\\ \left[\begin{array}{cc} -5 & -4 \end{array}\right] \end{array}\right)\right)$	$\left(\left(\begin{array}{c} \left[\begin{array}{cc} -7 & -5 \end{array}\right]\\ \left[\begin{array}{cc} -6 & -4 \end{array}\right]\\ \left[\begin{array}{cc} -9 & -3 \end{array}\right] \end{array}\right)\right)$

**Table 5:** For normalized NCq-ROFDM of *Q*_1_.

	*C*_1_	*C*_2_	*C*_3_	*C*_4_	*C*_5_
*A*_1_	$\left(\left(\begin{array}{c} \left[\begin{array}{cc} -5 & -4 \end{array}\right]\\ \left[\begin{array}{cc} -7 & -5 \end{array}\right]\\ \left[\begin{array}{cc} -7 & -2 \end{array}\right] \end{array}\right)\right)$	$\left(\left(\begin{array}{c} \left[\begin{array}{cc} -7 & -6 \end{array}\right]\\ \left[\begin{array}{cc} -3 & -2 \end{array}\right]\\ \left[\begin{array}{cc} -3 & -8 \end{array}\right] \end{array}\right)\right)$	$\left(\left(\begin{array}{c} \left[\begin{array}{cc} -5 & -3 \end{array}\right]\\ \left[\begin{array}{cc} -6 & -4 \end{array}\right]\\ \left[\begin{array}{cc} -6 & -8 \end{array}\right] \end{array}\right)\right)$	$\left(\left(\begin{array}{c} \left[\begin{array}{cc} -4 & -3 \end{array}\right]\\ \left[\begin{array}{cc} -3 & -2 \end{array}\right]\\ \left[\begin{array}{cc} -1 & -4 \end{array}\right] \end{array}\right)\right)$	$\left(\left(\begin{array}{c} \left[\begin{array}{cc} -6 & -3 \end{array}\right]\\ \left[\begin{array}{cc} -4 & -2 \end{array}\right]\\ \left[\begin{array}{cc} -8 & -1 \end{array}\right] \end{array}\right)\right)$
*A*_2_	$\left(\left(\begin{array}{c} \left[\begin{array}{cc} -3 & -2 \end{array}\right]\\ \left[\begin{array}{cc} -5 & -4 \end{array}\right]\\ \left[\begin{array}{cc} -8 & -2 \end{array}\right] \end{array}\right)\right)$	$\left(\left(\begin{array}{c} \left[\begin{array}{cc} -2 & -1 \end{array}\right]\\ \left[\begin{array}{cc} -7 & -6 \end{array}\right]\\ \left[\begin{array}{cc} -9 & -4 \end{array}\right] \end{array}\right)\right)$	$\left(\left(\begin{array}{c} \left[\begin{array}{cc} -7 & -5 \end{array}\right]\\ \left[\begin{array}{cc} -4 & -3 \end{array}\right]\\ \left[\begin{array}{cc} -5 & -8 \end{array}\right] \end{array}\right)\right)$	$\left(\left(\begin{array}{c} \left[\begin{array}{cc} -7 & -6 \end{array}\right]\\ \left[\begin{array}{cc} -2 & -1 \end{array}\right]\\ \left[\begin{array}{cc} -6 & -3 \end{array}\right] \end{array}\right)\right)$	$\left(\left(\begin{array}{c} \left[\begin{array}{cc} -2 & -1 \end{array}\right]\\ \left[\begin{array}{cc} -5 & -4 \end{array}\right]\\ \left[\begin{array}{cc} -7 & -4 \end{array}\right] \end{array}\right)\right)$
*A*_3_	$\left(\left(\begin{array}{c} \left[\begin{array}{cc} -9 & -7 \end{array}\right]\\ \left[\begin{array}{cc} -2 & -1 \end{array}\right]\\ \left[\begin{array}{cc} -6 & -1 \end{array}\right] \end{array}\right)\right)$	$\left(\left(\begin{array}{c} \left[\begin{array}{cc} -9 & -7 \end{array}\right]\\ \left[\begin{array}{cc} -2 & -1 \end{array}\right]\\ \left[\begin{array}{cc} -6 & -2 \end{array}\right] \end{array}\right)\right)$	$\left(\left(\begin{array}{c} \left[\begin{array}{cc} -8 & -6 \end{array}\right]\\ \left[\begin{array}{cc} -7 & -3 \end{array}\right]\\ \left[\begin{array}{cc} -8 & -5 \end{array}\right] \end{array}\right)\right)$	$\left(\left(\begin{array}{c} \left[\begin{array}{cc} -6 & -5 \end{array}\right]\\ \left[\begin{array}{cc} -7 & -5 \end{array}\right]\\ \left[\begin{array}{cc} -9 & -2 \end{array}\right] \end{array}\right)\right)$	$\left(\left(\begin{array}{c} \left[\begin{array}{cc} -6 & -4 \end{array}\right]\\ \left[\begin{array}{cc} -3 & -2 \end{array}\right]\\ \left[\begin{array}{cc} -6 & -5 \end{array}\right] \end{array}\right)\right)$
*A*_4_	$\left(\left(\begin{array}{c} \left[\begin{array}{cc} -5 & -3 \end{array}\right]\\ \left[\begin{array}{cc} -6 & -4 \end{array}\right]\\ \left[\begin{array}{cc} -7 & -4 \end{array}\right] \end{array}\right)\right)$	$\left(\left(\begin{array}{c} \left[\begin{array}{cc} -3 & -2 \end{array}\right]\\ \left[\begin{array}{cc} -8 & -5 \end{array}\right]\\ \left[\begin{array}{cc} -6 & -4 \end{array}\right] \end{array}\right)\right)$	$\left(\left(\begin{array}{c} \left[\begin{array}{cc} -6 & -5 \end{array}\right]\\ \left[\begin{array}{cc} -5 & -5 \end{array}\right]\\ \left[\begin{array}{cc} -5 & -3 \end{array}\right] \end{array}\right)\right)$	$\left(\left(\begin{array}{c} \left[\begin{array}{cc} -8 & -7 \end{array}\right]\\ \left[\begin{array}{cc} -9 & -5 \end{array}\right]\\ \left[\begin{array}{cc} -5 & -4 \end{array}\right] \end{array}\right)\right)$	$\left(\left(\begin{array}{c} \left[\begin{array}{cc} -4 & -2 \end{array}\right]\\ \left[\begin{array}{cc} -3 & -2 \end{array}\right]\\ \left[\begin{array}{cc} -5 & -4 \end{array}\right] \end{array}\right)\right)$

**Table 6:** Of normalized NCq-ROFDM of *Q*_2_.

	*C*_1_	*C*_2_	*C*_3_	*C*_4_	*C*_5_
*A*_1_	$\left(\left(\begin{array}{c} \left[\begin{array}{cc} -6 & -3 \end{array}\right]\\ \left[\begin{array}{cc} -5 & -4 \end{array}\right]\\ \left[\begin{array}{cc} -6 & -1 \end{array}\right] \end{array}\right)\right)$	$\left(\left(\begin{array}{c} \left[\begin{array}{cc} -7 & -3 \end{array}\right]\\ \left[\begin{array}{cc} -5 & -4 \end{array}\right]\\ \left[\begin{array}{cc} -9 & -4 \end{array}\right] \end{array}\right)\right)$	$\left(\left(\begin{array}{c} \left[\begin{array}{cc} -7 & -3 \end{array}\right]\\ \left[\begin{array}{cc} -5 & -4 \end{array}\right]\\ \left[\begin{array}{cc} -9 & -4 \end{array}\right] \end{array}\right)\right)$	$\left(\left(\begin{array}{c} \left[\begin{array}{cc} -9 & -6 \end{array}\right]\\ \left[\begin{array}{cc} -5 & -5 \end{array}\right]\\ \left[\begin{array}{cc} -4 & -1 \end{array}\right] \end{array}\right)\right)$	$\left(\left(\begin{array}{c} \left[\begin{array}{cc} -2 & -2 \end{array}\right]\\ \left[\begin{array}{cc} -9 & -5 \end{array}\right]\\ \left[\begin{array}{cc} -9 & -7 \end{array}\right] \end{array}\right)\right)$
*A*_2_	$\left(\left(\begin{array}{c} \left[\begin{array}{cc} -8 & -5 \end{array}\right]\\ \left[\begin{array}{cc} -7 & -6 \end{array}\right]\\ \left[\begin{array}{cc} -4 & -3 \end{array}\right] \end{array}\right)\right)$	$\left(\left(\begin{array}{c} \left[\begin{array}{cc} -6 & -2 \end{array}\right]\\ \left[\begin{array}{cc} -6 & -5 \end{array}\right]\\ \left[\begin{array}{cc} -6 & -1 \end{array}\right] \end{array}\right)\right)$	$\left(\left(\begin{array}{c} \left[\begin{array}{cc} -8 & -5 \end{array}\right]\\ \left[\begin{array}{cc} -6 & -3 \end{array}\right]\\ \left[\begin{array}{cc} -6 & -3 \end{array}\right] \end{array}\right)\right)$	$\left(\left(\begin{array}{c} \left[\begin{array}{cc} -6 & -2 \end{array}\right]\\ \left[\begin{array}{cc} -8 & -6 \end{array}\right]\\ \left[\begin{array}{cc} -6 & -3 \end{array}\right] \end{array}\right)\right)$	$\left(\left(\begin{array}{c} \left[\begin{array}{cc} -7 & -2 \end{array}\right]\\ \left[\begin{array}{cc} -4 & -5 \end{array}\right]\\ \left[\begin{array}{cc} -7 & -1 \end{array}\right] \end{array}\right)\right)$
*A*_3_	$\left(\left(\begin{array}{c} \left[\begin{array}{cc} -3 & -2 \end{array}\right]\\ \left[\begin{array}{cc} -5 & -5 \end{array}\right]\\ \left[\begin{array}{cc} -9 & -6 \end{array}\right] \end{array}\right)\right)$	$\left(\left(\begin{array}{c} \left[\begin{array}{cc} -6 & -5 \end{array}\right]\\ \left[\begin{array}{cc} -7 & -4 \end{array}\right]\\ \left[\begin{array}{cc} -6 & -1 \end{array}\right] \end{array}\right)\right)$	$\left(\left(\begin{array}{c} \left[\begin{array}{cc} -7 & -6 \end{array}\right]\\ \left[\begin{array}{cc} -7 & -4 \end{array}\right]\\ \left[\begin{array}{cc} -9 & -8 \end{array}\right] \end{array}\right)\right)$	$\left(\left(\begin{array}{c} \left[\begin{array}{cc} -8 & -6 \end{array}\right]\\ \left[\begin{array}{cc} -5 & -5 \end{array}\right]\\ \left[\begin{array}{cc} -6 & -4 \end{array}\right] \end{array}\right)\right)$	$\left(\left(\begin{array}{c} \left[\begin{array}{cc} -9 & -8 \end{array}\right]\\ \left[\begin{array}{cc} -6 & -5 \end{array}\right]\\ \left[\begin{array}{cc} -7 & -1 \end{array}\right] \end{array}\right)\right)$
*A*_4_	$\left(\left(\begin{array}{c} \left[\begin{array}{cc} -4 & -2 \end{array}\right]\\ \left[\begin{array}{cc} -8 & -5 \end{array}\right]\\ \left[\begin{array}{cc} -8 & -7 \end{array}\right] \end{array}\right)\right)$	$\left(\left(\begin{array}{c} \left[\begin{array}{cc} -9 & -4 \end{array}\right]\\ \left[\begin{array}{cc} -7 & -5 \end{array}\right]\\ \left[\begin{array}{cc} -6 & -6 \end{array}\right] \end{array}\right)\right)$	$\left(\left(\begin{array}{c} \left[\begin{array}{cc} -8 & -7 \end{array}\right]\\ \left[\begin{array}{cc} -6 & -5 \end{array}\right]\\ \left[\begin{array}{cc} -7 & -4 \end{array}\right] \end{array}\right)\right)$	$\left(\left(\begin{array}{c} \left[\begin{array}{cc} -6 & -2 \end{array}\right]\\ \left[\begin{array}{cc} -9 & -5 \end{array}\right]\\ \left[\begin{array}{cc} -5 & -4 \end{array}\right] \end{array}\right)\right)$	$\left(\left(\begin{array}{c} \left[\begin{array}{cc} -7 & -5 \end{array}\right]\\ \left[\begin{array}{cc} -6 & -4 \end{array}\right]\\ \left[\begin{array}{cc} -9 & -3 \end{array}\right] \end{array}\right)\right)$

**Table 7:** Of normalized NCq-ROFDM of *Q*_3_.

	*C*_1_	*C*_2_	*C*_3_	*C*_4_	*C*_5_
*A*_1_	$\left(\left(\begin{array}{c} \left[\begin{array}{cc} -4 & -2 \end{array}\right]\\ \left[\begin{array}{cc} -5 & -3 \end{array}\right]\\ \left[\begin{array}{cc} -7 & -1 \end{array}\right] \end{array}\right)\right)$	$\left(\left(\begin{array}{c} \left[\begin{array}{cc} -8 & -7 \end{array}\right]\\ \left[\begin{array}{cc} -4 & -2 \end{array}\right]\\ \left[\begin{array}{cc} -9 & -4 \end{array}\right] \end{array}\right)\right)$	$\left(\left(\begin{array}{c} \left[\begin{array}{cc} -4 & -1 \end{array}\right]\\ \left[\begin{array}{cc} -5 & -4 \end{array}\right]\\ \left[\begin{array}{cc} -2 & -6 \end{array}\right] \end{array}\right)\right)$	$\left(\left(\begin{array}{c} \left[\begin{array}{cc} -5 & -3 \end{array}\right]\\ \left[\begin{array}{cc} -4 & -2 \end{array}\right]\\ \left[\begin{array}{cc} -1 & -7 \end{array}\right] \end{array}\right)\right)$	$\left(\left(\begin{array}{c} \left[\begin{array}{cc} -6 & -3 \end{array}\right]\\ \left[\begin{array}{cc} -4 & -2 \end{array}\right]\\ \left[\begin{array}{cc} -6 & -3 \end{array}\right] \end{array}\right)\right)$
*A*_2_	$\left(\left(\begin{array}{c} \left[\begin{array}{cc} -6 & -4 \end{array}\right]\\ \left[\begin{array}{cc} -2 & -1 \end{array}\right]\\ \left[\begin{array}{cc} -3 & -5 \end{array}\right] \end{array}\right)\right)$	$\left(\left(\begin{array}{c} \left[\begin{array}{cc} -6 & -5 \end{array}\right]\\ \left[\begin{array}{cc} -4 & -3 \end{array}\right]\\ \left[\begin{array}{cc} -9 & -4 \end{array}\right] \end{array}\right)\right)$	$\left(\left(\begin{array}{c} \left[\begin{array}{cc} -4 & -2 \end{array}\right]\\ \left[\begin{array}{cc} -6 & -5 \end{array}\right]\\ \left[\begin{array}{cc} -7 & -7 \end{array}\right] \end{array}\right)\right)$	$\left(\left(\begin{array}{c} \left[\begin{array}{cc} -9 & -6 \end{array}\right]\\ \left[\begin{array}{cc} -5 & -3 \end{array}\right]\\ \left[\begin{array}{cc} -2 & -8 \end{array}\right] \end{array}\right)\right)$	$\left(\left(\begin{array}{c} \left[\begin{array}{cc} -2 & -1 \end{array}\right]\\ \left[\begin{array}{cc} -4 & -2 \end{array}\right]\\ \left[\begin{array}{cc} -7 & -2 \end{array}\right] \end{array}\right)\right)$
*A*_3_	$\left(\left(\begin{array}{c} \left[\begin{array}{cc} -2 & -1 \end{array}\right]\\ \left[\begin{array}{cc} -4 & -3 \end{array}\right]\\ \left[\begin{array}{cc} -9 & -6 \end{array}\right] \end{array}\right)\right)$	$\left(\left(\begin{array}{c} \left[\begin{array}{cc} -5 & -4 \end{array}\right]\\ \left[\begin{array}{cc} -3 & -2 \end{array}\right]\\ \left[\begin{array}{cc} -7 & -4 \end{array}\right] \end{array}\right)\right)$	$\left(\left(\begin{array}{c} \left[\begin{array}{cc} -2 & -1 \end{array}\right]\\ \left[\begin{array}{cc} -7 & -5 \end{array}\right]\\ \left[\begin{array}{cc} -3 & -8 \end{array}\right] \end{array}\right)\right)$	$\left(\left(\begin{array}{c} \left[\begin{array}{cc} -6 & -5 \end{array}\right]\\ \left[\begin{array}{cc} -7 & -5 \end{array}\right]\\ \left[\begin{array}{cc} -9 & -2 \end{array}\right] \end{array}\right)\right)$	$\left(\left(\begin{array}{c} \left[\begin{array}{cc} -7 & -4 \end{array}\right]\\ \left[\begin{array}{cc} -2 & -1 \end{array}\right]\\ \left[\begin{array}{cc} -6 & -5 \end{array}\right] \end{array}\right)\right)$
*A*_4_	$\left(\left(\begin{array}{c} \left[\begin{array}{cc} -5 & -3 \end{array}\right]\\ \left[\begin{array}{cc} -6 & -4 \end{array}\right]\\ \left[\begin{array}{cc} -5 & -5 \end{array}\right] \end{array}\right)\right)$	$\left(\left(\begin{array}{c} \left[\begin{array}{cc} -3 & -2 \end{array}\right]\\ \left[\begin{array}{cc} -8 & -5 \end{array}\right]\\ \left[\begin{array}{cc} -6 & -4 \end{array}\right] \end{array}\right)\right)$	$\left(\left(\begin{array}{c} \left[\begin{array}{cc} -5 & -3 \end{array}\right]\\ \left[\begin{array}{cc} -4 & -2 \end{array}\right]\\ \left[\begin{array}{cc} -4 & -5 \end{array}\right] \end{array}\right)\right)$	$\left(\left(\begin{array}{c} \left[\begin{array}{cc} -8 & -6 \end{array}\right]\\ \left[\begin{array}{cc} -8 & -5 \end{array}\right]\\ \left[\begin{array}{cc} -5 & -4 \end{array}\right] \end{array}\right)\right)$	$\left(\left(\begin{array}{c} \left[\begin{array}{cc} -5 & -2 \end{array}\right]\\ \left[\begin{array}{cc} -2 & -2 \end{array}\right]\\ \left[\begin{array}{cc} -5 & -6 \end{array}\right] \end{array}\right)\right)$

**Table 8:** Of normalized NCq-ROFDM of *Q*_4_.

	*C*_1_	*C*_2_	*C*_3_	*C*_4_	*C*_5_
*A*_1_	$\left(\left(\begin{array}{c} \left[\begin{array}{cc} -5 & -4 \end{array}\right]\\ \left[\begin{array}{cc} -7 & -5 \end{array}\right]\\ \left[\begin{array}{cc} -7 & -2 \end{array}\right] \end{array}\right)\right)$	$\left(\left(\begin{array}{c} \left[\begin{array}{cc} -7 & -6 \end{array}\right]\\ \left[\begin{array}{cc} -3 & -2 \end{array}\right]\\ \left[\begin{array}{cc} -3 & -8 \end{array}\right] \end{array}\right)\right)$	$\left(\left(\begin{array}{c} \left[\begin{array}{cc} -5 & -3 \end{array}\right]\\ \left[\begin{array}{cc} -6 & -4 \end{array}\right]\\ \left[\begin{array}{cc} -6 & -8 \end{array}\right] \end{array}\right)\right)$	$\left(\left(\begin{array}{c} \left[\begin{array}{cc} -4 & -3 \end{array}\right]\\ \left[\begin{array}{cc} -3 & -2 \end{array}\right]\\ \left[\begin{array}{cc} -1 & -4 \end{array}\right] \end{array}\right)\right)$	$\left(\left(\begin{array}{c} \left[\begin{array}{cc} -6 & -3 \end{array}\right]\\ \left[\begin{array}{cc} -4 & -2 \end{array}\right]\\ \left[\begin{array}{cc} -8 & -1 \end{array}\right] \end{array}\right)\right)$
*A*_2_	$\left(\left(\begin{array}{c} \left[\begin{array}{cc} -3 & -2 \end{array}\right]\\ \left[\begin{array}{cc} -5 & -4 \end{array}\right]\\ \left[\begin{array}{cc} -8 & -2 \end{array}\right] \end{array}\right)\right)$	$\left(\left(\begin{array}{c} \left[\begin{array}{cc} -2 & -1 \end{array}\right]\\ \left[\begin{array}{cc} -7 & -6 \end{array}\right]\\ \left[\begin{array}{cc} -9 & -4 \end{array}\right] \end{array}\right)\right)$	$\left(\left(\begin{array}{c} \left[\begin{array}{cc} -7 & -5 \end{array}\right]\\ \left[\begin{array}{cc} -4 & -3 \end{array}\right]\\ \left[\begin{array}{cc} -5 & -8 \end{array}\right] \end{array}\right)\right)$	$\left(\left(\begin{array}{c} \left[\begin{array}{cc} -7 & -6 \end{array}\right]\\ \left[\begin{array}{cc} -2 & -1 \end{array}\right]\\ \left[\begin{array}{cc} -6 & -3 \end{array}\right] \end{array}\right)\right)$	$\left(\left(\begin{array}{c} \left[\begin{array}{cc} -2 & -1 \end{array}\right]\\ \left[\begin{array}{cc} -5 & -4 \end{array}\right]\\ \left[\begin{array}{cc} -7 & -4 \end{array}\right] \end{array}\right)\right)$
*A*_3_	$\left(\left(\begin{array}{c} \left[\begin{array}{cc} -9 & -7 \end{array}\right]\\ \left[\begin{array}{cc} -2 & -1 \end{array}\right]\\ \left[\begin{array}{cc} -6 & -1 \end{array}\right] \end{array}\right)\right)$	$\left(\left(\begin{array}{c} \left[\begin{array}{cc} -9 & -7 \end{array}\right]\\ \left[\begin{array}{cc} -2 & -1 \end{array}\right]\\ \left[\begin{array}{cc} -6 & -2 \end{array}\right] \end{array}\right)\right)$	$\left(\left(\begin{array}{c} \left[\begin{array}{cc} -8 & -6 \end{array}\right]\\ \left[\begin{array}{cc} -7 & -3 \end{array}\right]\\ \left[\begin{array}{cc} -8 & -5 \end{array}\right] \end{array}\right)\right)$	$\left(\left(\begin{array}{c} \left[\begin{array}{cc} -6 & -5 \end{array}\right]\\ \left[\begin{array}{cc} -7 & -5 \end{array}\right]\\ \left[\begin{array}{cc} -9 & -2 \end{array}\right] \end{array}\right)\right)$	$\left(\left(\begin{array}{c} \left[\begin{array}{cc} -6 & -4 \end{array}\right]\\ \left[\begin{array}{cc} -3 & -2 \end{array}\right]\\ \left[\begin{array}{cc} -6 & -5 \end{array}\right] \end{array}\right)\right)$
*A*_4_	$\left(\left(\begin{array}{c} \left[\begin{array}{cc} -5 & -3 \end{array}\right]\\ \left[\begin{array}{cc} -6 & -4 \end{array}\right]\\ \left[\begin{array}{cc} -7 & -4 \end{array}\right] \end{array}\right)\right)$	$\left(\left(\begin{array}{c} \left[\begin{array}{cc} -3 & -2 \end{array}\right]\\ \left[\begin{array}{cc} -8 & -5 \end{array}\right]\\ \left[\begin{array}{cc} -6 & -4 \end{array}\right] \end{array}\right)\right)$	$\left(\left(\begin{array}{c} \left[\begin{array}{cc} -6 & -5 \end{array}\right]\\ \left[\begin{array}{cc} -5 & -5 \end{array}\right]\\ \left[\begin{array}{cc} -5 & -3 \end{array}\right] \end{array}\right)\right)$	$\left(\left(\begin{array}{c} \left[\begin{array}{cc} -8 & -7 \end{array}\right]\\ \left[\begin{array}{cc} -9 & -5 \end{array}\right]\\ \left[\begin{array}{cc} -5 & -4 \end{array}\right] \end{array}\right)\right)$	$\left(\left(\begin{array}{c} \left[\begin{array}{cc} -4 & -2 \end{array}\right]\\ \left[\begin{array}{cc} -3 & -2 \end{array}\right]\\ \left[\begin{array}{cc} -5 & -4 \end{array}\right] \end{array}\right)\right)$

**Table 9:** For collective NCq-ROFDM of M.

	*C*_1_	*C*_2_	*C*_3_	*C*_4_	*C*_5_
*A*_1_	$\left(\left(\begin{array}{c} \left[\begin{array}{cc} -882357 & -0100657 \end{array}\right]\\ \left[\begin{array}{cc} -722689 & -063629 \end{array}\right]\\ \left[\begin{array}{cc} -437647 & -078382 \end{array}\right] \end{array}\right)\right)$	$\left(\left(\begin{array}{c} \left[\begin{array}{cc} -677505 & -440853 \end{array}\right]\\ \left[\begin{array}{cc} -094596 & -0287674 \end{array}\right]\\ \left[\begin{array}{cc} -816469 & -176754 \end{array}\right] \end{array}\right)\right)$	$\left(\left(\begin{array}{c} \left[\begin{array}{cc} -156341 & -056971 \end{array}\right]\\ \left[\begin{array}{cc} -7804565 & -057936 \end{array}\right]\\ \left[\begin{array}{cc} -709723 & -048765 \end{array}\right] \end{array}\right)\right)$	$\left(\left(\begin{array}{c} \left[\begin{array}{cc} -980032 & -657461 \end{array}\right]\\ \left[\begin{array}{cc} -745276 & -045512 \end{array}\right]\\ \left[\begin{array}{cc} -832719 & -621549 \end{array}\right] \end{array}\right)\right)$	$\left(\left(\begin{array}{c} \left[\begin{array}{cc} -786541 & -004215 \end{array}\right]\\ \left[\begin{array}{cc} -967331 & -898736 \end{array}\right]\\ \left[\begin{array}{cc} -481265 & -343255 \end{array}\right] \end{array}\right)\right)$
*A*_2_	$\left(\left(\begin{array}{c} \left[\begin{array}{cc} -0637383 & -420758 \end{array}\right]\\ \left[\begin{array}{cc} -854671 & -542951 \end{array}\right]\\ \left[\begin{array}{cc} -0764617 & -032604 \end{array}\right] \end{array}\right)\right)$	$\left(\left(\begin{array}{c} \left[\begin{array}{cc} -976432 & -785421 \end{array}\right]\\ \left[\begin{array}{cc} -6432515 & -443045 \end{array}\right]\\ \left[\begin{array}{cc} -816469 & -176754 \end{array}\right] \end{array}\right)\right)$	$\left(\left(\begin{array}{c} \left[\begin{array}{cc} -156341 & -056972 \end{array}\right]\\ \left[\begin{array}{cc} -7804565 & -057936 \end{array}\right]\\ \left[\begin{array}{cc} -709723 & -048765 \end{array}\right] \end{array}\right)\right)$	$\left(\left(\begin{array}{c} \left[\begin{array}{cc} -844501 & -032167 \end{array}\right]\\ \left[\begin{array}{cc} -726235 & -692963 \end{array}\right]\\ \left[\begin{array}{cc} -564317 & -463246 \end{array}\right] \end{array}\right)\right)$	$\left(\left(\begin{array}{c} \left[\begin{array}{cc} -854156 & -064874 \end{array}\right]\\ \left[\begin{array}{cc} -905332 & -170456 \end{array}\right]\\ \left[\begin{array}{cc} -567812 & -462467 \end{array}\right] \end{array}\right)\right)$
*A*_3_	$\left(\left(\begin{array}{c} \left[\begin{array}{cc} -96319 & -580327 \end{array}\right]\\ \left[\begin{array}{cc} -494761 & -423218 \end{array}\right]\\ \left[\begin{array}{cc} -998348 & -257343 \end{array}\right] \end{array}\right)\right)$	$\left(\left(\begin{array}{c} \left[\begin{array}{cc} -049304 & -394847 \end{array}\right]\\ \left[\begin{array}{cc} -768512 & -126789 \end{array}\right]\\ \left[\begin{array}{cc} -346092 & -566718 \end{array}\right] \end{array}\right)\right)$	$\left(\left(\begin{array}{c} \left[\begin{array}{cc} -998601 & -266534 \end{array}\right]\\ \left[\begin{array}{cc} -599851 & -32192 \end{array}\right]\\ \left[\begin{array}{cc} -908723 & -231168 \end{array}\right] \end{array}\right)\right)$	$\left(\left(\begin{array}{c} \left[\begin{array}{cc} -304653 & -086215 \end{array}\right]\\ \left[\begin{array}{cc} -374209 & -174129 \end{array}\right]\\ \left[\begin{array}{cc} -444578 & -235075 \end{array}\right] \end{array}\right)\right)$	$\left(\left(\begin{array}{c} \left[\begin{array}{cc} -946115 & -386430 \end{array}\right]\\ \left[\begin{array}{cc} -753521 & -064251 \end{array}\right]\\ \left[\begin{array}{cc} -987801 & -8521133 \end{array}\right] \end{array}\right)\right)$
*A*_4_	$\left(\left(\begin{array}{c} \left[\begin{array}{cc} -643012 & -074213 \end{array}\right]\\ \left[\begin{array}{cc} -818596 & -254591 \end{array}\right]\\ \left[\begin{array}{cc} -303785 & -032105 \end{array}\right] \end{array}\right)\right)$	$\left(\left(\begin{array}{c} \left[\begin{array}{cc} -88506 & -873400 \end{array}\right]\\ \left[\begin{array}{cc} -246543 & -194085 \end{array}\right]\\ \left[\begin{array}{cc} -256375 & -019642 \end{array}\right] \end{array}\right)\right)$	$\left(\left(\begin{array}{c} \left[\begin{array}{cc} -970547 & -075908 \end{array}\right]\\ \left[\begin{array}{cc} -568652 & -181623 \end{array}\right]\\ \left[\begin{array}{cc} -960782 & -567149 \end{array}\right] \end{array}\right)\right)$	$\left(\left(\begin{array}{c} \left[\begin{array}{cc} -974534 & -375413 \end{array}\right]\\ \left[\begin{array}{cc} -568786 & -293648 \end{array}\right]\\ \left[\begin{array}{cc} -851636 & -166284 \end{array}\right] \end{array}\right)\right)$	$\left(\left(\begin{array}{c} \left[\begin{array}{cc} - & 26301-143665 \end{array}\right]\\ \left[\begin{array}{cc} -974624 & -356891 \end{array}\right]\\ \left[\begin{array}{cc} -708643 & -226138 \end{array}\right] \end{array}\right)\right)$

**Table 10:** Ranking result for various values of parameter *q*.

*Q*	Score values	Ranking results
*q*=4	*S*_1_=−.5378, *S*_2_=−.5479, *S*_3_=−.5248, *S*_4_=−.5406	${\overset{`}{A}}_{3}>A_{1}>A_{4}>A_{2}$
*q*=5	*S*_1_=−.5389, *S*_2_=−.5499, *S*_3_=−.5348, *S*_4_=−.5443	${\overset{`}{A}}_{3}>A_{1}>A_{4}>A_{2}$
*q*=7	*S*_1_=−.5225, *S*_2_=−.5489, *S*_3_=−.5129, *S*_4_=−.5460	${\overset{`}{A}}_{3}>A_{1}>A_{4}>A_{2}$
*q*=8	*S*_1_=−.5485, *S*_2_=−.5879, *S*_3_=−.5381, *S*_4_=−.5498	${\overset{`}{A}}_{3}>A_{1}>A_{4}>A_{2}$

**Table 11:** Ranking result for different values of parameters *j* and *k*.

j And k	Score values	Ranking results
j=0, k=1	S_1_=−.5286, S_2_=−.5759, S_3_=−.5148, S_4_=−.5463	A_3_ > A_1_ > A_4_ > A_2_
j=3, k=1	S_1_=−.5409, S_2_=−.5592, S_3_=−.5948, S_4_=−.5873	A_1_ > A_2_ > A_4_ > A_3_
j=1, k=3	S_1_=−.5825, S_2_=−.4489, S_3_=−.5879, S_4_=−.5260	A_2_ > A_4_ > A_1_ > A_3_
j=0, k=5	S_1_=−.5695, S_2_=−.5779, S_3_=−.5235, S_4_=−.5983	A_3_ > A_1_ > A_2_ > A_4_
j=5, k=6	S_1_=−.5805, S_2_=−.5949, S_3_=−.5621, S_4_=−.5498	A_4_ > A_3_ > A_1_ > A_2_
j=7, k=1	S_1_=−.5951, S_2_=−.5765, S_3_=−.5743, S_4_=−.5885	A_3_ > A_2_ > A_4_ > A_1_
j=0, k=3	S_1_=−.5195, S_2_=−.5669, S_3_=−.5930, S_4_=−.5573	A_1_ > A_4_ > A_2_ > A_3_
j=1, k=0	S_1_=−.4585, S_2_=−.5379, S_3_=−.3981, S_4_=−.5198	A_3_ > A_1_ > A_4_ > A_2_
j=5, k=5	S_1_=−.5578, S_2_=−.5678, S_3_=−.5421, S_4_=−.5950	A_3_ > A_1_ > A_2_ > A_4_
j=6, k=4	S_1_=−.5085, S_2_=−.3459, S_3_=−.4081, S_4_=−.4985	A_2_ > A_3_ > A_4_ > A_1_

## Data Availability

No data were used to support this study.
